The article "Dynamic Data Infrastructure Security for Interoperable e-Healthcare Systems: A Semantic Feature-Driven NoSQL Intrusion Attack Detection Model" was retracted in 2024. Reasons: signs of a paper mill; suspected computer-generated content; unreliable results or conclusions; concerns about the data.

# Dynamic Data Infrastructure Security for Interoperable e-Healthcare Systems: A Semantic Feature-Driven NoSQL Intrusion Attack Detection Model

**DOI:** 10.1155/2022/4080199

**Published:** 2022-06-10

**Authors:** R. Sreejith, S. Senthil

**Affiliations:** ^1^School of Computing and Information Technology, REVA University, Bangalore, India; ^2^School of Computer Science and Applications, REVA University, Bangalore, India

## Abstract

The exponential rise in advanced software computing and low-cost hardware has broadened the horizon for the Internet of Medical Things (IoMT), interoperable e-Healthcare systems serving varied purposes including electronic healthcare records (EHRs) and telemedicine. However, being heterogeneous and dynamic in nature, their database security remains a challenge forever. Numerous intrusion attacks including bot-attack and malware have confined major classical databases towards e-Healthcare. Despite the robustness of NoSQL over the structured query language databases, the dynamic data nature over a heterogeneous environment makes it vulnerable to intrusion attacks, especially over interoperable e-Healthcare systems. Considering these challenges, this work proposed a first of its kind semantic feature-driven NoSQL intrusion attack (NoSQL-IA) detection model for interoperable e-Healthcare systems. This work assessed the efficacy of the different semantic feature-extraction methods like Word2Vec, Continuous Bag of Words, N-Skip Gram (SKG), Count Vectorizer, TF-IDF, and GLOVE towards NoSQL-IA prediction. Subsequently, to minimize computational exhaustion, different feature selection methods including Wilcoxon Rank Sum Test (WRST), significant predictor test, principal component analysis, Select K-Best, and variance threshold feature selection algorithms were employed. To alleviate the data imbalance problem, it applied different resampling methods including upsampling, downsampling, and synthetic minority oversampling technique (SMOTE) over the selected features. Later, Min–Max normalization was performed over the input feature vectors to alleviate any possibility of overfitting. Towards NoSQL-IA prediction, different machine learning methods like Multinomial Naïve Bayes, decision tree, logistic regression, support vector machine, k-NN, AdaBoost, Extra Tree Classifier, random forest ensemble, and XG-Boost were applied, which classified each input query as the regular query or the NoSQL-IA attack query. The depth performance assessment revealed that the use of Word2Vec features SKG in sync with VTFS feature selection and SMOTE resampling processed with the bootstrapped random forest classifier can provide the best performance in terms of high accuracy (98.86%), F-Measure (0.974), and area under the curve (AUC) (0.981), thus enabling it suitable for interoperable e-Healthcare database security.

The article "Dynamic Data Infrastructure Security for Interoperable e-Healthcare Systems: A Semantic Feature-Driven NoSQL Intrusion Attack Detection Model" was retracted in 2024. Reasons: signs of a paper mill; suspected computer-generated content; unreliable results or conclusions; concerns about the data.

## 1. Introduction

The high-pace rise in technologies, especially software computing, cloud computing, and low-cost hardware technologies, has broadened the horizon for the different applications to make timely, decentralized, and accurate decisions. It has helped almost every socioeconomic and industrial segment to exploit aforesaid technologies towards optimal decision-making in query-driven services in business communication, industrial monitoring and control, finance, healthcare, science and technologies, education, entertainment, etc. The Healthcare sector has always remained a quality-concerned vertical demanding seamless communication to serve telemedicine, EHRs, e-medical, computer-aided diagnosis (CAD), health insurance services, etc. [1]. The benefits of online in healthcare involve unequalled speed and information availability, which can assist in overcoming the challenges that leading companies and patients confront. The cloud may aid in clinical trial governance and knowledge exchange, and this cutting-edge technology has altered the scope of clinical research [2, 3]. e-Health technologies comprise varied practices like sensory data collection and logging, electronic computer-aided diagnosis (e-CAD) and detail sharing, cloud data upload and decentralized data access for telemedicine, etc. [1, 4]. Noticeably, the aforesaid tasks often involve data communication and data logging to the decentralized cloud or central warehouses or databases [5, 6]. In today's healthcare system, there is a significant danger of data misinterpretation and inaccuracy. It is also inconvenient and takes time. As the number of patient and healthcare institutions has grown, traditional management practices have gone out of favor. As a result, a comprehensive healthcare management system has grown increasingly important over time [7, 8]. To cope up with e-Health demands, interoperable systems provide a platform(s) for multiple stakeholders like patients, doctors, hospital management, lab technicians, nurses, and guardians with their corresponding roles, rights, and access provision [9, 10]. In this manner, the different users can have other notions, intends, intelligible inputs, and distinct writing structures, giving rise to a heterogeneous data environment with the databases. Under such a complex data environment identifying a malicious intruder turns out to be a challenge [5, 6]. Despite the fact that providing an interoperable framework can provide “Fit-To-All” solution for e-Healthcare, however, guaranteeing data security would always remain a challenge [5]. The recent events of unauthorized data breaches caused billions of dollars due to unauthorized insurance claims and patients' personal details for the different monitory benefits [5]. It has alarmed industries to ensure healthcare data security. Towards healthcare data security, different methods like steganography, cryptosystems, and blockchain have been proposed [1, 4]; however, the recent attacks like brute force, smart card loss, and impersonation have confined major solutions [10, 11]. Most of the existing methods have focused on encryption; however, very few efforts are made towards “data infrastructure security” [11]. Though different databases or allied data infrastructures employ gate-level access control using certain authentication methods, however, the nature of intrusion attacks often makes them inferior (see Section 2). This is because the hackers often intrude inside databases by mimicking genuine data structures or injecting malicious codes at the place of query variables [12–15].

e-Health makes use of a number of digital technologies. Users of e-Health can use the Internet to communicate with healthcare workers over e-mail, access medical records, research health information, and share text, audio, video, and other data [16, 17]. Polycom, or mobile TV, facilitates audio and video communications between two or more individuals in two or more locations. Kiosks in e-Health are self-contained devices (usually PCs) that provide interactive information to users [18, 19]. Interoperable e-Healthcare services apply databases in the form of local data warehouses or cloud storage to enable decentralized query-driven decision support [5, 6]. The intrusion risk turns out to be more severe with dynamic data storage and access ecosystem where the different users of the different types may use it for real-time decision-making [5]. In sync with EHRs or the patient's healthcare records (PHRs), the different users can make an access request or data log or even online computation on the same data infrastructure. The processes involve data feed, query-driven data retrieval, and online computation and update, hence, making them dynamic in nature. Moreover, there can be different e-Healthcare terminals like wireless body area networks, wearable healthcare devices, quantified-self devices, and web-based applications where the data can be logged or updated dynamically [4]. Most of the classical databases use certain relational database management approaches, which are often characterized in terms of their fixed or static schema, vertical scalability, etc. (i.e.., SQL). However, being vertical in nature, the classical SQL-driven relational databases struggle in delivering fast responses especially over large inputs [5, 6]. To cope with time-efficient and interoperable system demands, NoSQL databases, which are often characterized in the form of their robust dynamic structure, hierarchical data storage, and vertical scalability, have gained widespread attention [9, 10]. Their efficacy in coping with more complex queries to serve real-time EHRs or telemedicine purposes makes them suitable for interoperable e-Healthcare [13]. NoSQL databases like MongoDB and CouchDB, Key-value: Redis and DynamoDB, Wide-column: Cassandra and HBase, and Graph: Neo4j and Amazon Neptune are found more efficient in terms of availability, credibility, identification, and automatic functional capabilities [13]. Such robustness makes NoSQL a suitable database candidate for a time-efficient and scalable solution towards interoperable e-Healthcare [11]. Despite all these advantages, the possibility and challenges of infiltration attacks in NoSQL cannot be ruled out [11]. Being an interoperable e-Healthcare system with multiple stakeholders, the data input and allied characteristics can be different that consequently making classical intrusion detection methods inappropriate [13, 14]]. The classical term-matching-based intrusion detection methods might fail in detecting the malicious user or query [12–14]. Miscalculation towards the wrongly classified queries can force the model to under false-positive performance and hence can impact reliability. Noticeably, so far almost all existing intrusion detection systems focused on SLI-intrusion attack (SQLIA) detection, and no significant effort has been made toward intrusion detection in NoSQL databases [14]. This, as a result, broadens the gaps for academia industries to develop a robust intrusion detection system for NoSQL dynamic datasets for e-Healthcare systems [12, 14]. An intrusion detection system (IDS) is a software application that detects network intrusions using machine learning algorithms. IDS monitors a network or system for malicious behavior and protects against unauthorized access from users, including insiders [15, 20].

The article "Dynamic Data Infrastructure Security for Interoperable e-Healthcare Systems: A Semantic Feature-Driven NoSQL Intrusion Attack Detection Model" was retracted in 2024. Reasons: signs of a paper mill; suspected computer-generated content; unreliable results or conclusions; concerns about the data.

Considering at hand solutions, merely syntactic analysis and term-matching cannot be suitable for NoSQL-IA prediction. It can give rise to false-positive performance with reduced reliability. Classical manual testing methods are limited to identifying intrusion attacks in large databases with multiple stakeholders over interoperable designs [11]. To cope with intrusion detection demands over the heterogeneous and dynamic data-based e-Healthcare system, developing a universal query learning and decision system (UQLDS) can be vital. Moreover, applying machine intelligence to understand each query from multiple sources is a must, and therefore, this problem can be well solved using natural learning programming. NLP can help understand different kinds of queries with varied structures or schema. However, unlike SQLIA, the efficacy of the NoSQL-IA detection model would mainly depend on the efficacy of the features being learnt and the algorithms being applied [14]. In addition to the suitable set of features, it also requires identifying the set of robust computational ecosystems armored with information-rich feature extraction method(s), computation-centric feature selection followed by highly efficient classification to perform reliable intrusion detection [5]. Unlike classical SQLIA methods employing query mapping and structural analysis, NoSQL-IA detection requires semantic feature learning ability [10]. Extracting semantic features from dynamic queries (at both gate level as well as within database transactions), one can apply machine learning models to identify the intrusion attack. However, identifying the optimal set of algorithms, including feature engineering and classification is a must for NoSQL-IA prediction [10]. In addition to the semantic feature need, NoSQL-IA detection model requires addressing the class-imbalance problem as well. This is because the number of intrusions in a real-time environment is always smaller in volume in the minority and therefore training a machine learning over the majority class can skew the prediction results (i.e., false-positive result). Though different machine learning algorithms have been applied towards intrusion detection, yet generalizing one's superiority is difficult due to diversity in their performance over the different test cases. Therefore, it is vital to assess varied machine learning methods and identify the best approach for the NoSQL-IA model. Generally, the telemedicine ecosystem is heterogeneous concerning data, storage, and data transfer methods. Intrusion detection models are typically deployed at the application level, which gives the privilege of scalability and context switching concerning the application environment. The proposed model focuses on constructing a semantic feature-driven intrusion detection system exploring the possibility of natural language processing, text mining, and machine learning. It is always possible to switch to a model trained with SQLIA dataset, which makes the system to adapt the heterogeneity of the telemedicine application environment.

In sync with above discussed key challenges and allied scopes, in this paper, a robust NoSQL-IA detection model is developed for interoperable e-Healthcare systems. The proposed NoSQL-IA detection focuses on improving feature superiority and computing robustness to achieve optimal performance. The proposed model applies different semantic feature extraction methods like Word2Vec, Continuous Bag of Word (CBOW), GLOVE, Skip-N-Gram (SKG), and Count Vectorizer (COUTV) towards their suitability for the NoSQL-IA model. Once extracting these semantic features, different feature selection methods were applied, including WRST, significant predictor test (SPT), principal component analysis (PCA), Select K-Best (SKB), and variance threshold feature selection (VTFS) algorithms. Here, the key motive was to assess which specific feature and allied feature selection method is effective for NoSQL-IA prediction. The bootstrap method is a common resampling technique that uses replacement sampling to estimate statistics on a population. If the data contains a small number of extreme values, bootstrapping will undervalue these observations as bias correction is not performed. Bootstrap will not be very accurate if the samples are not representative of the entire population. Instead of duplicate data points, SMOTE creates synthetic data points that deviate slightly from the original data points. This method creates a representative sample from the minority group. As the data cannot fully represent the population in the research scenario, the proposed method is applied to alleviate the class-imbalance problem. Subsequently, the selected features were processed for Min–Max normalization to alleviate the overfitting problem. The relationship between the original data values is preserved with Min–Max normalization. In our scenario, we use Min–Max normalization as there is a high chance the data distribution may not be Gaussian, and the feature always falls within a bounded interval. Finally, the input features were processed for two-class classification using different algorithms including Multinomial Naïve Bayes (MNB), decision tree (DT), logistic regression (LOGR), AdaBoost (ADAB), Extra Tree Classifier (ETC), random forest (RF), and XG-Boost classifier. Here, the key motive was to identify the best performing classifier for NoSQL-IA prediction. The overall proposed model was assessed over NoSQL (MongoDB database retrieved from interoperable system design), and data revealed that the proposed NoSQL-IA model exhibits superior performance in terms of accuracy, F-Measure, and area under the curve (AUC) results. Some of the key contributions of this research are given as follows:

Key Contributions:

- This work is the first of its kind effort towards intrusion detection in dynamic data structures like NoSQL for interoperable e-Healthcare services. Unlike classical SQLIA detection methods, especially term-matching or structural analysis approaches, NoSQL-IA model exploited semantic features derived from input queries to train the model that enabling it to achieve higher accuracy and reliability even under dynamic data structures. Here, semantic feature learning helped in coping with the dynamic data structure
- Realizing “query-driven features” as the backbone towards intrusion prediction, this work applied advanced feature engineering methods including semantic feature extraction, feature selection, data resampling, and normalization, along with state-of-the-art novel heterogeneous ensemble classification. This cumulative solution helped accomplish a reliable and highly accurate model for NoSQL-ID detection
- Though there are numerous feature extraction methods and hence to identify the optimally performing features, four different feature extraction methods like Word2Vec, CBOW, N-Skip Gram, Count Vectorizer, GLOVE, and TF-IDF were applied. Here, the key purpose was to identify the best performing feature towards NoSQL-IA detection
- In sync with time and computation efficient NoSQL-IA detection, the proposed model applied different feature selection methods including PCA, WRST, VTFS, and SKB heuristic algorithms. Similar to the feature extraction methods, this work examines the relative efficacy of the different feature selection methods towards NoSQL-IA detection
- Unlike major existing injection attack detection approaches which often ignore the class-imbalance problem in intrusion detection, this work exploited multiple resampling techniques including UPS, DPS, and SMOTE to assess their efficacy to achieve superior NoSQL-IA detection
- In the real-time dynamic data structure, especially under interoperable e-Healthcare systems operating environment, the nonlinearity of the input data might force machine learning algorithm(s) to undergo convergence and overfitting problems. To alleviate these problems, the proposed model performs Min–Max normalization over the inputs (i.e., selected resampled features). It helps achieve better computation with superior learning
- The proposed NoSQL-IA model assessed different machine learning classifiers to identify the best suitable model for NoSQL-IA prediction
- Finally, the overall proposed model identifies the set of the best performing feature extraction, feature selection, resampling, and machine learning methods towards NoSQL-IA prediction. Thus, the eventual model provides a robust computing environment for NoSQL-IA prediction, which can be applied for intrusion detection at both “gate-level” security as well as “within data infrastructure” security
- Amongst the different sets of features and allied computing environment, this research identified that word-embedding methods like Word2Vec and SKG could be vital with WRST feature selection, SMOTE resampling, and RF classifier. This eventual set of the computing environment can be vital towards NoSQL-IA prediction

The other sections of this manuscript are divided as follows. Section 2 discusses the background of the interoperable e-Healthcare system and intrusion scopes.  Section 3 presents the related works, followed by research questions and problem formulation in Section 4.  Section 5 presents the proposed model implementation, which is followed by results and discussion in Section 6.  Section 7 presents the conclusion. References used in this manuscript are given at the end of the manuscript.

The article "Dynamic Data Infrastructure Security for Interoperable e-Healthcare Systems: A Semantic Feature-Driven NoSQL Intrusion Attack Detection Model" was retracted in 2024. Reasons: signs of a paper mill; suspected computer-generated content; unreliable results or conclusions; concerns about the data.

## 2. NoSQL Injection Threat in Interoperable e-Healthcare Systems

In the majority of the interoperable services including the e-Healthcare, humongous amount of data is generated from the different users having different purposes, intends, and taxonomies. Such systems often give rise to or undergo heterogeneous data environments where the applications often intend to provide query-driven analytics support swiftly with high intelligibility and accuracy. To cope up with such demands, NoSQL databases have gained widespread attention serving a large amount of cloud-based or even ERP-driven solutions serving numerous industrial verticals. Unlike classical SQL databases, NoSQL or not only SQL databases are characterized in the form of horizontal structure with superior time efficiency, availability, and high scalability. Such robustness makes it suitable towards interoperable services like e-Healthcare software systems or services. However, unlike SQL query structure which is fixed in nature, the dynamic nature of NoSQL makes it more vulnerable towards intrusion attacks. Similar to the other databases, NoSQL too undergoes allied functions like data creation, update, reading, and deletion. In the case of interoperable e-Healthcare services or software as well, the different stakeholders including patients, doctors, attendants, laboratory staff, and even insurance agents can have access to their respective data for real-time decision-making. To perform their respective job(s), the stakeholders often employ a function called a query. For query-driven tasks, databases provide a dedicated input box that enables different users to input the intended or expected data, details, etc. These input queries can be for both data retrieval as well as upload or update and hence undergoes continuous transaction during the operating period. While developing the system, the interoperable systems or allied functions store the inputs and allied variables used in the query. These input variables can be numbers, letters, data sequences containing notations, etc., in each query (say, query statement). These variables are employed to execute certain predefined tasks or functions. However, in case such variables are not assessed before executing any task, it can cause disaster in the form of intrusion attacks, manipulations, data deletion, etc. Here, the key threat is that the intruder or the malicious code would be executed once the query is running. Such intrusion can cause data manipulation, data bypass, data deletion, and sometimes encryption to cause ransomware attacks. Therefore, any possibility of such intrusion can be dangerous for databases including NoSQL, which itself is dynamic and heterogeneous in nature under interoperable applications. Same as SQL statement segmentation, intrusion, or malicious codes can change the functions in NoSQL databases like MongoDB. An illustration of the query statements in the SQL and NoSQL (MongoDB) database is depicted in Figure 1. This query intends to retrieve patient-related information.

The article "Dynamic Data Infrastructure Security for Interoperable e-Healthcare Systems: A Semantic Feature-Driven NoSQL Intrusion Attack Detection Model" was retracted in 2024. Reasons: signs of a paper mill; suspected computer-generated content; unreliable results or conclusions; concerns about the data.

Observing Figure 1, it can be easily found that the intruders or hackers might write and execute malicious codes and maybe feed them to the query's input boxes to get executed. This process is often called intrusion. Though attackers cannot inject complete arbitrary code, they can still set up attacks by injecting unvalidated inputs and using a small set of functions.

For example, the code below fetches the record with the name (attribute) ‘Mr.Bean' using the $where query operator.

Secure Coding Practices, Least Privilege Policy, and Input Validation are the most common techniques to prevent NoSQL injections in practice. Along with Input Validation, the proposed NoSQL-IA model enables application-level security to avoid data breaches and access breaches. Since overcomplex and multistakeholder driven interoperable models like e-Healthcare systems, the intrusion query or malicious code can be put into the condition statement directly, it becomes easier for hackers to retrieve information by executing injection easily (say, successfully). The severity of such intrusion can be higher in the case of interoperable e-Healthcare systems where the query elements or variables by the different users can be different from each other. For instance, a doctor writes a prescription or diagnosis decisions in the different medicine-related taxonomy or words; on the contrary, a patient with average language ability can feed any comfortable word(s) to state its condition or query. Such heterogeneity might broaden the gap for hackers to intrude or inject intrusion attacks successfully. This, as a result, makes the overall database system vulnerable, and, therefore, there is the need for a robust NoSQL-IA detection model which could have the ability to learn to intend, scope and highly intrinsic information from each query to detect an attack or allied malicious code. It can be considered as the key driving force behind this study.

The article "Dynamic Data Infrastructure Security for Interoperable e-Healthcare Systems: A Semantic Feature-Driven NoSQL Intrusion Attack Detection Model" was retracted in 2024. Reasons: signs of a paper mill; suspected computer-generated content; unreliable results or conclusions; concerns about the data.

## 3. Related Work

A major fraction of the recently developed machine learning-driven intrusion detection models has focused on SQL intrusion attack (SQLIA) detection. For instance, SEPTIC, a machine learning-driven SQLIA model, was developed in [21], yet it underwent high false positive due to a low feature quotient in structural information used for training. Despite exploiting deep features in [22–24], the authors failed to achieve efficient performance towards intrusion detection. The key limitation of this approach was the lack of ability to address the class imbalance and heterogeneous data processing (ability). Deep learning and allied features were applied in [21] as well towards SQLIA. Authors [25] inferred that under dynamic data conditions, intrusion detection could be solved as an NLP problem rather than syntax matching or term-matching stereotypes. To improve feature efficiency, the authors [26] suggested using Word2Vec word-embedding concept for injection detection in databases. Authors [27] made an effort to improve feature information as well as learning by means of an adaptive deep-forest model; however, in addition to the increased computational complexity and exhaustion, AdaBoost-based classifier could exhibit low accuracy (near 90%), signifying high false-positive results. Despite an effort towards a multilevel regular expression paradigm to perform SQLIA prediction, authors [28] failed to achieve higher accuracy over dynamic data. Moreover, this approach was suitable mainly for static databases like SQL or XML. Authors in [29, 30] developed a penetrating testing-driven attack detection or intrusion detection model. However, its ability towards nonlinear, heterogeneous traffic remains suspicious. Authors in [31] revealed that the inferior SQL query's structural information forces machine learning models to undergo increased false positive, especially under dynamic databases like a web-interfaced database. Similar inferences can be observed towards (SQL) query-manipulation detection-based methods, especially under dynamic run-time systems [32]. Though, in [22, 33], the authors suggested exploiting high-dimensional features extracted from the SQL queries to perform SQLIA, yet, their relevance towards NoSQL databases remains an unexplored domain. Despite a vital effort towards SQLIA prediction, authors failed to address their suitability over dynamic data structures such as NoSQL datasets, especially under heterogeneous data inputs. In [34], recently, authors developed a semantic feature-driven consensus-based learning environment for SQLIA prediction; however, it failed to address heterogeneous and distributed dynamic data learning, which is quite more complex than the classical static databases like SQL. The model trained with static database structure like SQL cannot be generalized over distributed dynamic databases like NoSQL [12–14]. The authors proposed case-based reasoning (CBR) engine equipped with learning and adaptation capacity for SQLIA. However, the accuracy of 93.8% doesn't guarantee its suitability with dynamic data because of its higher reliance on the predefined structural information-driven learning ability. Moreover, the lack of class-imbalance solutions in major machine learning-driven methods like [35] results in reduced and nongeneralizable outcomes [36]. Author [37] applied syntax-structure learning concept towards injection detection; however, lower computational efficiency (accuracy 83.1%) confines it is more limited for NoSQL databases. Noticeably, these approaches cannot be suitable for NoSQL databases due to dynamic data in nature and different data structures [38]. Authors in [39] applied Two-Class SVM (TC SVM) and Two-Class LR (TC LR) towards injection attack detection using Microsoft Azure Machine Learning (MAML) in online systems. Naïve Bayes (NB) algorithm was applied in [39] to perform a role-based access control and injection attack. Recently, authors [40] found that for dynamic data analysis and allied intrusion prediction, semantic features such as SKG can be of vital significance. Despite numerous efforts, above stated methods are assessed with fixed data structure, and hence, their suitability towards heterogeneous, nonlinear data (say, dynamic data structure) seems limited. However, the key suggestions or allied inferences obtained from these intrusion detection methods indicate that the use of semantic features can be more effective, while addressing key challenges like class imbalance and data heterogeneity can help achieve superior performance towards intrusion detection in real-time databases.

The article "Dynamic Data Infrastructure Security for Interoperable e-Healthcare Systems: A Semantic Feature-Driven NoSQL Intrusion Attack Detection Model" was retracted in 2024. Reasons: signs of a paper mill; suspected computer-generated content; unreliable results or conclusions; concerns about the data.

Unlike SQLIA, recently, a few efforts were made toward NoSQL intrusion detection. For instance, authors [41] developed an intrusion detection model for MongoDB and CouchDB, which are well-known and highly used NoSQL databases. Authors [42] applied One-class SVM (OC-SVM) to perform intrusion detection over NoSQL databases. However, neither it could exploit semantic feature efficacy nor even address computational improvement as a goal toward generalizable performance. Similar to [43], authors in [42] developed a Bayesian network as a K2 algorithm for intrusion detection in MongoDB NoSQL-IA detection. However, the basic computational environment broadens the horizon for further study and innovation. In [43], the authors applied different machine learning methods for intrusion detection in MongoDB databases. Despite multiple machine learning models, this study inferred that the random forest method could be superior to classical k-NN, DT, and Naïve Bayes (NB) algorithms. Despite RF-based classification, this approach failed to address semantic feature significance, class-imbalance problems, etc., which can limit its efficacy towards real-time interoperable system design [44, 45]. Authors [41] found that the major interoperable systems developed onto JavaScript development platforms (specially designed with MongoDB databases) are susceptible to intrusion attacks; however, merely applying syntax features and code review cannot yield an optimal detection solution. Authors in [46] developed Diglossia, a sophisticated tool for intrusion attack detection over SQL and NoSQL queries. In order to detect intrusion attacks, their proposed model parses the inputs or queries and assesses whether the two parse trees are syntactically isomorphic. In [47], the authors developed an intrusion detection system for two well-known NoSQL datasets, Cassandra and MongoDB. Yet, their efficacy remained limited to real-time interoperable system designs. Authors in [48] discussed security concerns, especially over decentralized Hadoop has driven NoSQL databases and stated that to cope with the different intrusion attack detection demands, developing a query-learning concept can be vital rather than predefined rule-based methods. Authors in [49] suggested a reversible watermarking-based security model for NoSQL data security. However, it merely focuses on data security based on unique embedding features and does not guarantee any intrusion-related attack scenario. Though authors in [50] developed a NoSQL intrusion detection method, yet it failed to exploit semantic features and advanced computing methods for NoSQL-IA detection. The depth assessment of the different existing approaches reveals that towards intrusion detection, merely applying syntactic information or structural rule learning cannot yield reliable intrusion detection in a real-time system, and hence, semantic features can yield more superior performance towards intrusion attack detection in databases [34, 39–41, 43]. Moreover, in addition to semantic feature learning, improving the computational environment with advanced feature selection, resampling, and classification is a must. Moreover, assessing the suitability of the aforesaid methods also needed to be tested with dynamic distributed data with interoperable heterogeneous query elements [51–53]. These key factors can be considered the key driving forces behind this study.

The article "Dynamic Data Infrastructure Security for Interoperable e-Healthcare Systems: A Semantic Feature-Driven NoSQL Intrusion Attack Detection Model" was retracted in 2024. Reasons: signs of a paper mill; suspected computer-generated content; unreliable results or conclusions; concerns about the data.

## 4. Problem Formulation

The key challenge in an interoperable system e-Healthcare system is data security and reliability. In such an interoperable system, there can be multiple user types with distinct roles, rights, and access credentials. In such systems, the data patterns can be heterogeneous and can be more severe with e-Healthcare systems [5, 6, 9–12]. Under such a heterogeneous and complex working environment, assessing each input query or allied appropriateness is challenging. Considering such adversity and allied scopes, different intruders often make use of intrusion attacks to get access to the databases to perform data manipulation, alteration, deletion, etc. In addition to these, the cases of ransomware attacks to being witnessed globally, where an intruder mimics the normal queries and enters the database to manipulate access or data sources. In classical SQL databases, which are static, identifying intrusion is relatively easier due to the static query nature and syntactic comparison ability. However, almost all major SQL-driven databases are time-consuming and hence undergo delay over real-time interoperable system demands. Moreover, merely applying query-matching or syntactic analysis cannot guarantee intrusion detection because the recent intrusion efforts have been applying sophisticatedly designed bots that mimic the original queries and hence detecting them based on structure or syntax turns out to be infeasible. It infers that both the classical SQL data structures and allied intrusion detection models are limited to addressing contemporary attack scenarios, malicious code, or bot-driven attacks. To alleviate these problems, dynamic data structures such as NoSQL have gained widespread attention [12–14]. Their dynamic data structure and interoperable characteristics make the system have superior availability, credibility, and time efficiency. Such robustness can help e-Healthcare systems, especially EHRs and telemedicine, to serve real-time demands. To be noted, being interoperable, the likelihood of attacks increases significantly over distributed dynamic data structures where the different users can input the different inputs having diverse intentions, terms, and meanings. In such a case, most of the existing intrusion detection methods can be limited due to low perceptibility and lack of universal intelligibility. Despite the robustness of NoSQL data structures towards interoperable data services, the attack likelihood remains the same with NoSQ- distributed data structure and hence requires a robust intrusion detection model which could identify the attacker query at both “at the gateway” as well as “within humongous database.” To achieve it, unlike classical text mining approaches, syntax matching, and keyword search methods, there is the need to upgrade the intelligibility of the detection model with more semantic information capacity. In other words, improving intrusion detection systems with more diverse semantic and latent information and allied traceability can help identify or classify intrusion queries accurately. Moreover, towards a large distributed framework like “interoperable e-Healthcare system,” applying manual testing approaches cannot be effective, and hence, it requires certain artificial intelligence-driven analytics solutions which could exploit the different distributed data structures and allied queries to build a superior intelligible knowledge bank for real-time intrusion tracking. To achieve it, unlike term frequency matching or syntactic analysis, semantic feature-driven machine learning models specially designed in sync with the natural language programming (NLP) paradigm can be vital [34, 54]. In sync with aforesaid semantic features, the use of machine learning model(s) can be vital to perform automatic intrusion detection in NoSQL distributed data structures toward secure, interoperable e-Healthcare systems. The proposed work is a kind of industry-level semantic feature-driven IDS focusing on NoSQL-IA for telemedicine applications. Additionally, the model of IDA shall be added to the existing telemedicine application server to enhance security at the application level. Also, the model can be considered as a security layer to the newly designed telemedicine framework.

The article "Dynamic Data Infrastructure Security for Interoperable e-Healthcare Systems: A Semantic Feature-Driven NoSQL Intrusion Attack Detection Model" was retracted in 2024. Reasons: signs of a paper mill; suspected computer-generated content; unreliable results or conclusions; concerns about the data.

Considering above stated research goals and allied scopes, in this paper, a first of its kind NoSQL-IA detection model is developed for distributed data structures to be used for interoperable e-Healthcare systems. The overall proposed model has been designed as an NLP problem where at first semantic features have been extracted from queries originating from the different interoperable sources (or stakeholders). Realizing the diversity of performance by the different feature extraction models, in this paper, four well-known semantic feature extraction methods named Word2Vec, CBOW, SKG, TF-IDF, Count Vectorizer, and GLOVE were applied that generate features distinctly. Subsequently, realizing the computational efficiency, the proposed model applies four different feature selection methods, including significant predictor test, WRST, PCA, VTFS, and SKB methods. Noticeably, these different feature selection algorithms are applied distinctly over the different features to assess the suitability of the dominant feature for NoSQL-IA prediction. Unlike major existing machine learning-based intrusion prediction models that often fail in addressing class-imbalance problems, the proposed model applies different resampling concepts to prepare feature vectors that sufficiently distribute minority as well as majority class data or events. It can help provide sufficiently large heterogeneous features to perform accurate NoSQL-IA prediction. Thus, once resampling input (selected) features, the proposed model applies Min–Max normalization to alleviate any possible overfitting or convergence problem. Finally, the normalized features were processed for classification using several state-of-the-art robust classifiers such as Multinomial Naïve Bayes, logistic regression, k-NN, decision tree, AdaBoost, Extra Tree Classifier, random forest, and XGBoost classifiers. Here, the key motive was to identify the best performing machine learning environment for NoSQL-IA prediction. Thus, applying above stated approach, the proposed model intends to perform “gate-level” as well “within database” intrusion detection to ensure the safety and security of the interoperable e-Healthcare systems for seamless decision-making. The overall research intends to achieve answer(s) for the following key research questions:

RQ1: Can the use of semantic features enable intrusion detection and classification in distributed data structures like NoSQL for interoperable e-Healthcare services?

RQ2: Which semantic feature extraction model be an optimally effective approach toward NoSQL-IA prediction in interoperable e-Healthcare services?

RQ3: Which feature resampling model be an optimally effective approach towards NoSQL-IA prediction in interoperable e-Healthcare services?

RQ4: Which machine learning model is optimally effective towards NoSQL-IA prediction in distributed data structures based on interoperable e-Healthcare services?

RQ5: What should be the set of a computing environment including feature extraction, selection, sampling, and classification to yield optimally accurate and reliable NoSQL-IA prediction for interoperable e-Healthcare services?

## 5. System Model

As discussed in the previous sections, the proposed NoSQL-IA prediction model is developed as an NLP problem where the key motive is to exploit semantic features from each query of the data entry and learn over a highly robust computing environment to classify it as normal or the NoSQL-IA attack query class. To achieve it, the proposed model applies phased implementation encompassing the following steps:

1. Data acquisition and preprocessing
2. Semantic feature extraction
3. Feature selection
4. Feature resampling
5. Feature normalization
6. NoSQL-IA classification

A detailed discussion of these key methods is given in the subsequent sections.

The article "Dynamic Data Infrastructure Security for Interoperable e-Healthcare Systems: A Semantic Feature-Driven NoSQL Intrusion Attack Detection Model" was retracted in 2024. Reasons: signs of a paper mill; suspected computer-generated content; unreliable results or conclusions; concerns about the data.

### 5.1. Data Acquisition and Preprocessing

In sync with the targeted interoperable e-Healthcare services using NoSQL databases and allied infrastructure security, the proposed model was specially designed for NoSQL databases. Undeniably, the majority of the interoperable e-Healthcare services and allied databases can be characterized in terms of heterogeneity and dynamic nature that makes intrusion detection a challenging task. On the other hand, the efficacy of intrusion detection models primarily depends on feature information and allied statistical characteristics (of the training datasets). Exploring in-depth, we observed that though a few benchmark datasets are available for SQL intrusion attack detection; however, there is no benchmark available for NoSQL-IA detection. Moreover, attack-annotation is a challenge in NoSQL-IA prediction. Considering this fact, we prepared our training dataset to validate the efficacy of the proposed NoSQL-IA prediction model toward interoperable e-Healthcare services. The considered data environment was distributed dynamically in nature with data heterogeneity, which is generated by the multiple users with different roles, meanings, and terminologies; a dynamic application was created. In the considered interoperable system environment, multiple users could interact with each other as well as with the system. In addition, the deployed system environment inculcated a static application as well, which does not possess any user and executes a static process each time to introduce a query to the system's database. This model of query execution was applied to introduce attack traces inside the database. A snippet of the data synthesis model developed is given in Figure 2.

Being distributed dynamically in nature, the proposed data environment resembles MongoDB and CouchDB, which can be characterized in the form of a NoSQL-Map database. For the proposed distributed dynamic data synthesis, the experimental setup discussed in Figure 2 was applied. The deployed approach enabled the generation of the different queries or traces towards NoSQL-IA prediction. The NoSQL-IA system has two significant entities, the trigger model and the serving infrastructure. As the system uses the containership concept of serving the model, the system is highly scalable concerning model upgradation and architecture expansion. When the telemedicine application scales up, the NoSQL-IA IDA shall have multiple containers synchronizing with any container orchestration tool of that particular server environment. The container is a lightweight virtualization technology similar to VM for creating isolated environments. Docker virtualizes applications, decouples them from their underlying devices, and allows them to be deployed and migrated between physical devices with ease. The proposed research uses Docker containers to simulate multiple instances and construct an isolated environment for model deployment. Kubernetes orchestration methods are explored to run the Docker containers. To alleviate any possibility of interferences over the interoperable framework (amongst the different users), a Docker container was deployed that was running over the MongoDB server in conjunction with a virtual machine setup (see VM1 in Figure 2). As depicted in Figure 2, Sysdig is executed within a kernel space and is functional towards call traces retrieval where the call traces are being generated by the running container. Here, in order to inculcate dynamic behavior with heterogeneous inputs (amongst the different interoperable users concurrently), the proposed model sent requests to the container by means of VM1 (Figure 2). To achieve this, the Apache JMeter workload generator tool was applied. Though a simple HTTP sampler of Apache JMeter can be applied on CouchDB to enable web traffic simulating different users, the study explores the possibility of Nmap and Metasploit tools for intrusion-related traces executed by VM2. In this work, JMeter with JSR223 sampler was applied to generate the traffic traces from the different users. Functionally, web requests were transmitted to the server to initiate the database functions. In sync with interoperable (system) functionality, for each application, two threads (i.e., Thread-1 and Thread-2 in JMeter) were deployed to send a request to the server simulation and post the data values concurrently. In the deployed platform, Thread-1 encompassed a total of 100 users that performed simultaneous document queries (say, enquiry) and (basic) data feed over the execution period. Similarly, Thread-2 encompassed four users (here, we hypothesized them to be doctors, hospital management, assistants, and lab technicians) having the right to create, update, and delete the database(s). Noticeably, in the deployed framework, as Apache JMeter generates the dynamic data traffic, Sysdig (Figure 2) performs monitoring of the queries or calls of the server, signifying the normal traces. In this work, we generated a total of 4000 traces with 347 intrusion traffic traces. Thus, collecting this database, we deployed it for feature engineering for further NoSQL-IA prediction tasks. Towards preprocessing task, the proposed model applied tokenization of the input queries, followed by stemming and stopping word's removal from making data suitable for feature generation. Once obtaining the token information for each query, the extracted data or tokens (per query) were processed for semantic feature extraction. The details of the proposed feature engineering model are given in the subsequent sections.

The article "Dynamic Data Infrastructure Security for Interoperable e-Healthcare Systems: A Semantic Feature-Driven NoSQL Intrusion Attack Detection Model" was retracted in 2024. Reasons: signs of a paper mill; suspected computer-generated content; unreliable results or conclusions; concerns about the data.

### 5.2. Semantic Feature Extraction

Being heterogeneous in nature, the collected query traces possessed varied tokens, operators, structural indexes, literals, punctuations, and identifiers. In addition, unlike classical structural query languages, the proposed dynamic distributed data NoSQL traces contains different clauses, predicates, and expressions. In such dynamic data structure and allied representation, assessing the hidden embedding information and allied semantic features can be of great significance towards NoSQL-IA prediction. In the input queries, the aforesaid clause, predicate, and expressions are employed to characterize a query to make further real-time NoSQL-IA predictions. Any intruding query can be strategically designed to mimic and penetrate normal NoSQL data structure in certain tautological types to retrieve outputs from a database far beyond the developer's intention. In NoSQL-IA, the sophistically designed attackers identify the poorly coupled clauses, predicates, and expressions due to dynamic structure to intrude inside. Though such specific structural features can be applied to static SQLIA; however, their generalization over dynamic data structure seems unrealistic. In the targeted distributed dynamic structure models, the specially designed bots can mimic the original query, and hence, intrusion becomes easier over dynamic (and heterogeneous) databases. Therefore, unlike classical structural features or syntax characteristics, this research work proposes to exploit semantic (or latent) features for the NoSQL-IA prediction task. Despite the fact that the semantic features can provide superior learning over classical structure-learning-based methods, different algorithms claim their superiority over others. Considering this motive, four different kinds of semantic feature extraction algorithms have been applied. These algorithms are:

1. Word2Vec word-embedding
2. N-Skip Gram method
3. Continuous Bag of Words (CBOW),
4. Count Vectorizer
5. GLOVE
6. TF-IDF

In the proposed work, the input queries or data samples are in the form of textual data, which is required to be encoded into relevant numeric vectors toward the corresponding feature representation. Considering this motive, the proposed model applied the concept of word-embedding that transforms input tokens or queries into related numeric (high-dimensional) feature presentations. This work applied the Word2Vec word-embedding concept that hypothesizes that the contexts in the natural presentation or language possess high correlation, and hence, the tokens (or words) can be vectorized as per the corresponding context. Subsequently, the word vector can be retrieved from the training corpus so as to measure the semantic similarity between different words (present in the natural language). In the proposed work, each processed token was converted into a numeric feature representation called a feature vector. Here, the Gensim Word2Vec model was designed with a double-layered neural network possessing two hidden layers, which helped to retain more sparse and significantly important features. Though Word2Veec is realized in two distinct configurations, CBOW and SKG, we applied these two methods to extract semantic features distinctly. A snippet of these algorithms is given as follows.

The article "Dynamic Data Infrastructure Security for Interoperable e-Healthcare Systems: A Semantic Feature-Driven NoSQL Intrusion Attack Detection Model" was retracted in 2024. Reasons: signs of a paper mill; suspected computer-generated content; unreliable results or conclusions; concerns about the data.

#### 5.2.1. N-Skip Gram (SKG)

Let the total set of words be {1, ⋯, *W*}. Then for a given NoSQL query set, the proposed Word2Vec N-Skip Gram method performs learning over the vector representation of each encompassing token *w*. In this manner, the obtained feature representations are processed for training to identify the words having a higher probability of taking place within the context window of a particular center word. In this manner, with the extracted input tokens from the query corpus (*w*_1_, ⋯, *w*_*T*_), the proposed model improves the probability of the context word in sync with the center word. Here, the prime motive was defined as

(1) $$\begin{array}{c} \overset{T}{\underset{t=1}{\sum }}\underset{c\in C_{t}}{\sum }\log p\left(w_{c}\;|\;w_{t}\right). \end{array}$$

In (1), *C*_*t*_ represents the factor called context window, which is decided around the centre token *w*_*t*_. In this manner, the probability of occurrence of the context word near the center word *w*_*t*_ is obtained as per the Softmax over the function defined in

(2) $$\begin{array}{c} p\left(w_{c}\;|\;w_{t}\right)=\frac{e^{s\left(w_{c}\;|\;w_{t}\right)}}{\sum_{j=1}^{W}e^{s\left(w_{t},j\right)}}. \end{array}$$

In (2), the parameter *s* signifies the scoring function representing the convolution of the centre word *w*_*t*_ and the corresponding context word. In this manner, an objective function *J*_*θ*_ (3) which is supposed to be reduced over training is defined.

(3) $$\begin{array}{c} J_{\theta }=-\underset{w_{i}\in V}{\sum }\log\frac{p\left(w_{i}\;|\;c\right)}{p\left(w_{i}\;|\;c\right)+kQ\left(w_{i}\right)}+\overset{k}{\underset{j=1}{\sum }}\log\frac{p\left({\bar{w}}_{i}\;|\;c\right)}{p\left({\bar{w}}_{ij}\;|\;c\right)+kQ\left({\bar{w}}_{ij}\right)}. \end{array}$$

In (3), *Q* states the noise distributions to be used for generating *k*-noise samples. The proposed work employed the embedding matrices obtained in reference to each *n*-gram in *n*-gram vocabulary to retrieve context words. In addition, we applied a token-only embedding matrix configured with *n* = 1, the window size of five long with the Skip Gram size of one. In our proposed model, each batch of input corpus, along with the labels passed over each run, transforms allied mapping output to the *n*-gram. It helped estimate the embedding vectors that eventually constitute required word vector representations. These word vectors were transformed to the loss function in which it applied SGDM (stochastic gradient descent model) to update embedding metrics. Updated embedding metrics were obtained as a feature vector for further processing.

The article "Dynamic Data Infrastructure Security for Interoperable e-Healthcare Systems: A Semantic Feature-Driven NoSQL Intrusion Attack Detection Model" was retracted in 2024. Reasons: signs of a paper mill; suspected computer-generated content; unreliable results or conclusions; concerns about the data.

#### 5.2.2. Word2Vec CBOW

A few existing pieces of literature criticize that N-Skip Gram methods often generate high-dimensional features increasing the computational complexity of the system. Unlike the N-Skip Gram method, CBOW Word2Vec methods provide more significant semantic features than NLP methods. In the CBOW method, the context token is predicted on the basis of the neighboring context-window. Now, let *W*_*i*−1_, *W*_*i*−2_, *W*_*i*+1_, *W*_*i*+2_ be the context word or corpus obtained from each NoSQL query, and then the proposed method predicts *W*_*i*_ that possesses a higher correlation with the other tokens in the corpus or query. The two distinct word-embedding sets of the native CBOW method are the source and target sides, signifying *v*_*w*_.*v*_*w*_′ ∈ ℝ^*d*^ for each token of the NoSQL query (i.e., *w* ∈ *V*). In this manner, a text-window can have the centre word *w*_0_ and the corresponding context words *w*_1_, ⋯, *w*_*C*_. Thus, for a predefined text-window representing a NoSQL query, we defined CBOW loss as

(4) $$\begin{array}{c} v_{c}=\frac{1}{C}\overset{C}{\underset{j=1}{\sum }}v_{w_{j}}, \end{array}$$

(5) $$\begin{array}{c} L=-\log\sigma \;\left(v_{w0}^{\prime }\;T_{v_{c}}\right)-\overset{k}{\underset{i=1}{\sum }}\log\sigma \left(-v_{n_{i}}^{\prime }\;T_{v_{c}}\right). \end{array}$$

In (5), the variable *n*_1_ ⋯ *n*_*k*_ ∈ *V* be the negative samples retrieved from the noise-distribution *P*_*n*_ over query corpus *V*. In (5), the gradient of *ℒ* in reference to the different components like the expected value *v*_*w*0_′, a negative target sample *v*_*n*_*i*__′ and average context source (*v*_*c*_) are represented as per ((6)–(8)), respectively.

(6) $$\begin{array}{c} \frac{\partial L}{\partial v_{w0}^{\prime }}=\left(\sigma \left(v_{w0}^{\prime }\;T_{v_{c}}\right)-1\right)v_{c}, \end{array}$$

(7) $$\begin{array}{c} \frac{\partial L}{\partial v_{n_{i}}^{\prime }}=\left(\sigma \left(v_{n_{i}}^{\prime }\;T_{v_{c}}\right)-1\right)v_{\text{c}}, \end{array}$$

(8) $$\begin{array}{c} \frac{\partial L}{\partial v_{c}}=\left(\sigma \left(v_{w0}^{\prime }\;T_{v_{c}}\right)-1\right)v_{w0}^{\prime }+\overset{k}{\underset{i=1}{\sum }}\left(\sigma \left(v_{n_{i}}^{\prime }\;T_{v_{c}}\right)-1\right)v_{n_{i}}^{\prime }. \end{array}$$

In this manner, employing the concept of chain rule with respect to the source context embedding, we obtained the feature vector as output (9).

(9) $$\begin{array}{c} \frac{\partial L}{\partial v_{w_{j}}}=\frac{1}{C}\left[\left(\sigma \left(v_{w0}^{\prime }\;T_{v_{c}}\right)-1\right)v_{w0}^{\prime }+\overset{k}{\underset{i=1}{\sum }}\left(\sigma \left(v_{n_{i}}^{\prime }\;T_{v_{c}}\right)-1\right)v_{n_{i}}^{\prime }\right]. \end{array}$$

Thus, for a given context window, say bag-of-words, it generates embedding metrics representing the semantically connected probable words, which are used for further training. In the CBOW feature extraction method, a key challenge is an incorrect update in the context vector, and, therefore, to alleviate it, we performed context word normalization. For context word normalization, we resampled the width of the context window randomly in the range of 1 to *C*_max_ for each target word. It broadened the context-embedding over the wider context window and provided more significant features for training.

The article "Dynamic Data Infrastructure Security for Interoperable e-Healthcare Systems: A Semantic Feature-Driven NoSQL Intrusion Attack Detection Model" was retracted in 2024. Reasons: signs of a paper mill; suspected computer-generated content; unreliable results or conclusions; concerns about the data.

#### 5.2.3. GLOVE

Different kinds of literature reveal that a superior word-embedding requires representing the words in such a manner that two distinct tokens or words possessing the same semantic inference or significance would have the same vector representations. In this manner, one can preserve the other linguistic associations amongst the varied words for better training. Similar to the above discussed Word2Vec word-embedding method(s), the approach called Global Vectors (GLOVE) is also a statistical unsupervised learning concept. However, unlike aforesaid methods, GLOVE exploits cooccurrence metrics to generate the numerical vector-space representation. In practice, it is accomplished by estimating how frequently the different words cooccur within a defined context window in a given query corpus. Subsequently, it applies the dimensional-reduction method over the cooccurrence matrix. Noticeably, based on the size of corpus employed for training, GLOVE method might demand significantly large memory, which can later make feature extraction and allied classification more exhaustive. However, to assess relative performance towards NoSQL-IA prediction, we employed the GLOVE method as one of the semantic feature extraction tools. To implement it, we employed a pretrained GLOVE model, which has been trained over the data corpora from Wikipedia and Gigaword. The pretrained model was prepared over the dataset encompassing a total of six billion tokens with a total vocabulary of 400,000 distinct words. In our proposed model, we considered the length of the vectorized word representation as 100, which helped reduce computational exhaustion in comparison to TF-IDF or classical Count Vectorizer.

#### 5.2.4. TF-IDF

Similar to the above-discussed GLOVE model, the TF-IDF method calculates the total number of the frequently occurred word identified based on the (frequent) occurrence of the words in a corpus. In our proposed NoSQL-IA detection model, TF-IDF was applied as a feature extraction model where it estimated the frequency of the term(s) within each query or input corpus. In the proposed feature extraction model, term frequency (TF) provides the total number of repeats that a specific word undergoes in the provided query or input corpus. It estimated the total number of repeats that a specific word does (within a provided input corpus) than the total number of tokens or words available in the input corpus. TF is estimated as per

(10) $$\begin{array}{c} {tf}_{i,j}=\frac{n_{ij}}{\sum_{k}n_{ij}}. \end{array}$$

In inverse data frequency (IDF), it calculated the number of occurrences of a unique token across the input corpus. Noticeably, tokens with very rare presence over an input corpus used to have larger IDF, which is obtained using

(11) $$\begin{array}{c} df\left(w\right)=\log\left(\frac{N}{{df}_{i}}\right). \end{array}$$

In this manner, applying the score over (10) and (11), scores, TF-IDF estimated a cumulative score value (*w*) for a token within an input query or allied corpus, using

(12) $$\begin{array}{c} w_{i,j}={t\text{f}}_{i,j}\times \log\left(\frac{N}{{df}_{i}}\right). \end{array}$$

In (12), *tf*_*i*,*j*_ represents the total number of occurrences of *i*-token in *j*th corpus. On the contrary, the number of queries possessing *i*-token is *df*_*i*_. Here, *N* represents the total number of queries. Once obtaining the TF-IDF score for each input token, the proposed model performed text-to-sequence conversion and thus estimated an equivalent sequence of words or values for further learning towards NoSQL-IA prediction.

The article "Dynamic Data Infrastructure Security for Interoperable e-Healthcare Systems: A Semantic Feature-Driven NoSQL Intrusion Attack Detection Model" was retracted in 2024. Reasons: signs of a paper mill; suspected computer-generated content; unreliable results or conclusions; concerns about the data.

In addition to the above-discussed feature extraction methods, we also applied Count Vectorizer (COUTV) using SciKit Learn Library in Python to extract features from the input queries. However, due to space constraints, a detailed discussion of COUTV is not given in this manuscript. The details of COUTV can be found in [49, 50].

### 5.3. Feature Selection

This is a matter of the fact that the above-stated word-embedding methods obtain high-dimensional information-rich feature sets for better learning, however, at the cost of increased search (or data) space and hence higher computational cost. In sync with real-time NoSQL-IA prediction demands, to alleviate this problem, in this paper, feature selection was performed. Here, the key motive was to reduce the insignificant or relatively low significant features to improve computational efficiency as well as better training. Different researches advocate different feature selection methods and, therefore, to identify the optimally performing feature set towards NoSQL-IA prediction. In this reference, the proposed model applies four different types of feature selection methods, including the following:

1. Select K-Best
2. Principal component analysis
3. Wilcoxon Rank Sum Test (WRST)
4. Variance threshold method

The detailed discussion of the overall proposed feature selection method is given as follows:

#### 5.3.1. Select K-Best Feature Selection

In this work, we applied SKB feature selection method that estimates the top-k most significant features. In our proposed Select K-Best-based feature selection, we applied the chi-squared method which helped in estimating the set of most significant features. A snippet of the proposed chi-squared SKB feature selection method is given as follows:

*(1) Univariate Chi-Squared Test*. The univariate chi-squared approach applies a criteria-driven feature selection concept where it estimates the vitality of a feature element by estimating *χ*^2^ statistics in reference to the target class. Here, each feature is examined for its vitality distinctly to assess the corresponding relationship to the target variable. It functions as a key nonparametric test approach to compare multiple variables for randomly selected data. Being a kind of the independence-test method, the proposed model enabled identifying the disparity and independence amongst multiple random variables. In this manner, it estimated a value based on the relationship between the feature instance and the class it should belong. For the out value 0, it states that there is no relationship between the feature element and the class. The higher association value shows a stronger relationship between the feature element and the class it should belong. Here, we employed the chi-squared concept towards initial feature estimation using SciKit Learn Library. Functionally, the chi-square's statistics approach is applied as per the information-theoretic feature selection paradigm. In this approach, it tries to assess the intuition that the term *t*_*k*_ for a specific label or class *c*_*i*_ is the one distributed amongst the set of positive and negative examples. Mathematically, the chi-squared test is defined as

(13) $$\begin{array}{c} Chi–Square\left(t_{k},c_{i}\right)=\frac{N{\left(AD-CB\right)}^{2}}{\left(A+C\right)\left(B+D\right)\left(C+D\right)}. \end{array}$$

In (13), *N* states the total number of feature elements in the corpus, while *A* states the elements in class *c*_*i*_ encompassing *t*_*k*_. The number of feature elements containing *t*_*k*_ in other classes is given by *B*, while the number of feature elements in class *c*_*i*_ which do not have any terms of *t*_*k*_ be *C*. The other parameter *D* states the number of feature elements having no term *t*_*k*_ in other classes. In this manner, applying (13), the proposed approach assigned a score for each feature towards each class (here, normal query or the NoSQL-IA query). Finally, the total scores are combined to give rise a final score, defined as

(14) $$\begin{array}{c} \max\left(Chi–Square\left(t_{k},c_{i}\right)\right). \end{array}$$

Thus, applying above method, we obtained the set of most significant features for further NoSQL-IA prediction task.

The article "Dynamic Data Infrastructure Security for Interoperable e-Healthcare Systems: A Semantic Feature-Driven NoSQL Intrusion Attack Detection Model" was retracted in 2024. Reasons: signs of a paper mill; suspected computer-generated content; unreliable results or conclusions; concerns about the data.

#### 5.3.2. Principal component analysis

To implement PCA, we calculated the principal component and eigenvalues of the covariance or correlation for each feature element. The distance between each feature element from the average principal component (here, 0.5) is considered here. Thus, those feature elements fulfilling this condition were retained for further computing. The selected feature elements were hypothesized to have a higher impact on prediction results. Those feature elements with a distance lower than the average principal component value of 0.5 were dropped from the further computation. In this manner, it helped retain only statistically significant feature elements to perform better learning and reduce redundant processing costs. The finally selected feature elements were used for further resampling and NoSQL-IA prediction or allied classification.

#### 5.3.3. Wilcoxon Mann–Whitney Test

This method is also called the significant predictor test. Wilcoxon Mann–Whitney Test also called Wilcoxon Rank Sum Test (WRST) is a kind of nonparametric test with independent samples. It assesses the correlation between the feature elements and their likelihood of NoSQL-IA prediction accuracy. Here, WRST was applied to estimate the correlation between the feature elements and allied corresponding class labels to perform NoSQL-IA prediction. The extracted feature elements are hypothesized to be the independent variable; on the contrary, the likelihood of NoSQL-IA is taken as the dependent variable. This approach enabled estimating the *p* value for each data element with respect to the corresponding significance towards NoSQL-IA probability, and therefore, employing the *p* value of each feature element, it labeled each data element as significant or insignificant. It helped identify a set of samples having an impact on NoSQL-IA probability and allied accuracy. It helped retain only those significant feature elements which had a significant impact on NoSQL-IA prediction.

The article "Dynamic Data Infrastructure Security for Interoperable e-Healthcare Systems: A Semantic Feature-Driven NoSQL Intrusion Attack Detection Model" was retracted in 2024. Reasons: signs of a paper mill; suspected computer-generated content; unreliable results or conclusions; concerns about the data.

#### 5.3.4. Variance Threshold Feature Selection

The variance threshold method is a baseline concept for feature selection. The ability to eliminate those feature elements whose variance does not fulfill some predefined or expected threshold makes it a goal-oriented feature selection approach. It assumes that the feature elements with high variance can have more significant information to make prediction. In this reference, in our work, the variance threshold method dropped all zero-variance feature elements (the feature elements with the same value in all samples). Unlike correlation test-based methods, the employed variance threshold method does not consider any correlation or relationship between features. We considered variance threshold as 0, signifying features with zero-variance, and therefore, identifying the feature elements with zero-variance, it dropped those specific feature elements and retained the set of feature elements with nonzero variance for further processing. Thus, applying these four feature selection methods, the suitable set of feature elements was retained for further computation.

### 5.4. Feature Resampling

This is a matter of the fact that the above-stated feature selection methods retained the optimal set of (distinct) features for NoSQL-IA training; however, the fact that the likelihood of NoSQL-IA intrusion query would be significantly lower than the normal query cannot be denied. In other words, in real-time NoSQL-IA data traces, the fraction of intrusion query is significantly lower than the normal queries, signifying the inevitable probability of class imbalance (or skewed data). Training a machine learning model over the skewed data or the class-imbalance training dataset can force the model to exhibit false-positive or skewed performance. To alleviate this problem, feature resampling can be of great significance. Towards feature resampling, the key methods used are random sampling, upsampling and downsampling. However, these methods have their own strengths as well as limitations. For instance, in random sampling, the samples from the minority class are selected arbitrarily and added to the original sample to increase the minority sample in the training set. Similarly, in UPS methods, the minority samples are increased using a certain method to reach uniform sample distribution. On the contrary, in DPS, the majority of samples are reduced to make minority samples sufficient for training. However, these approaches often give rise to the unbalanced data condition, which can impact NoSQL-IA prediction results. In this work, we performed resampling in such a manner that the minority samples are augmented with 95% of a confidence interval. We performed random duplication of the observations taken from the minority class that helped reinforce their respective values. However, such methods with sample duplication can give rise to iterative overfitting problems, and hence, we applied sampling strategy (SS), also called threshold adaptive sampling, to resample the input features. We applied *SS* = 0.5. In this case, for a case of 500 majority class samples and 50 minority samples, it inculcated 250 minority samples to the original feature set. Here, our key motive was to increase the number of minority class samples to provide fairly sufficient examples for training. To further improve the performance and data efficacy, we applied SMOTE as one of the resampling methods. We generated synthetic positive samples using the k-NN algorithm. We applied 5-nearest neighborhood to the minority “NoSQL-IA” class, which was followed by equalization of the samples in such a manner that it yields the number of the majority class same as the number of the minority class. Thus, in this work, a total of three resampling methods, including upsampling, downsampling, and SMOTE sampling, were applied distinctly over the selected features to assess the suitability of the best performance sampling method. The resampled outputs were processed for normalization so as to alleviate any possibility of overfitting.

The article "Dynamic Data Infrastructure Security for Interoperable e-Healthcare Systems: A Semantic Feature-Driven NoSQL Intrusion Attack Detection Model" was retracted in 2024. Reasons: signs of a paper mill; suspected computer-generated content; unreliable results or conclusions; concerns about the data.

### 5.5. Feature Normalization

In this paper, we applied Min–Max normalization over each feature set that mapped each input value to the scale of 0 to 1. Here, the Min–Max normalization algorithm, as defined in (15), mapped each data element in the range of [0-1]. It was achieved by transforming input features into the range of 0-1, linearly. The input data element *x*_*i*_ from feature element *X* was mapped to achieve the normalized value *x*_*i*_′ using (15). Here, min(*X*) and max(*X*) represents the minimum and maximum values of  *X*, correspondingly.

(15) $$\begin{array}{c} Norm\left(x_{i}\right)=x_{i}^{\prime }=\frac{x_{i}-\min\left(X\right)}{\max\left(X\right)-\min\left(X\right)}. \end{array}$$

As depicted in Table 1, post normalization, a total of 12 feature sets were obtained with respect to the different input features. These features were processed for two-class classification using the different machine learning methods. The details of the classification methods used in this work are given as follows:

### 5.6. NoSQL-IA Classification

Unlike classical standalone classifier-based learning, in this work, we applied an ensemble learning-assisted consensus-based classification model. Being a two-class classification problem, each classifier classifies the data and labels it as 1 or 0, signifying NoSQL-IA query and normal query, respectively. In this work, a total of seven well-known machine learning classifiers were used to perform NoSQL-IA prediction or allied classification. These machine learning models are:

1. Naïve Bayes Algorithm (NB)
2. Support vector machine (SVM)
3. Decision tree (DT)
4. Logistic regression (LOGR)
5. k-NN (KN)
6. AdaBoost (ADAB)
7. Random forest (RF)
8. Extra Tree Ensemble Classifier (ETC)
9. XGBoost (XGB)

A brief of these machine learning classifiers is given in the subsequent sections.

#### 5.6.1. Naïve Bayes Algorithm

Naïve Bayes is one of the predominantly used probabilistic classification approaches that apply Bayes' rules with autonomous assumptions to classify input patterns. Being a probabilistic approach, it is also stated as an “independent feature model” which assumes that all allied features are independent and do not impact result decisively. It assumes that the existence of a particular feature in a class is not related to the presence of another feature. Functionally, the NB algorithm allocates an object *x* to the class *e*^∗^ = argmax_d_P(d | x) as per the Bayes′ rule.

(16) $$\begin{array}{c} P\left(d\;|\;x\right)=\frac{P\left(x\;|\;d\right)P\left(d\right)}{P\left(x\right)}. \end{array}$$

In (16), *P*(*d*) refers to the class-prior probability of c. The other parameter *P*(*d* | *x*) states the likelihood of *x* data element, while *P*(*x*) states the predictor prior probability and is defined as

(17) $$\begin{array}{c} P\left(x\;|\;d\right)=\overset{m}{\underset{l=1}{\prod }}P\left(x_{l}\;|\;d\right). \end{array}$$

We applied a multinomial NB algorithm that, unlike Gaussian NB, learns on the basis of the count's frequency, signifying the number of times *x*_*i*_ occurs over *n* trails. Here, feature vectors state the frequency with which a specific event is caused by a multinomial function. NB algorithms classify each query as a normal query or NoSQL-IA query and label it as “0” and “1,” respectively.

The article "Dynamic Data Infrastructure Security for Interoperable e-Healthcare Systems: A Semantic Feature-Driven NoSQL Intrusion Attack Detection Model" was retracted in 2024. Reasons: signs of a paper mill; suspected computer-generated content; unreliable results or conclusions; concerns about the data.

#### 5.6.2. Support Vector Machine (SVM)

SVM represents a kind of supervised learning approach for pattern mining and classification. The ability to learn and categorize input patterns based on the hyperplane makes it one of the most suitable algorithms for text classification, image processing, etc. Functionally, it learns over the input features and functions as nonprobabilistic binary classifier. To perform NoSQL-IA prediction, SVM reduces the generalization error over the unobserved input patterns, often called instances. To achieve it, it applied a structural risk reduction method. In this approach, support vector refers the training instances or the set of training data that calculates the hyperplane between the two or multiple types of data patterns to perform classification. To achieve it, it employs

(18) $$\begin{array}{c} Y^{\prime }=w*\phi \left(x\right)+b. \end{array}$$

In (18), *ϕ*(*x*) states the nonlinear transform where it focuses on assigning the suitable values of the weight *w* and the bias *b* values to perform classification. The output Y′ is estimated by reducing the regression-risk parameter, given as

(19) $$\begin{array}{c} R_{reg}\left(Y^{\prime }\right)=C*\overset{l}{\underset{i=0}{\sum }}\gamma \left(Y_{i}^{\prime }-Y_{i}\right)+\frac{1}{2}*{\left\|w\right\|}^{2}. \end{array}$$

In equation (19), *C* presents the penalty factor, while the cost function is *γ*. We estimated the weight value using

(20) $$\begin{array}{c} w=\overset{l}{\underset{j=1}{\sum }}\left(\alpha_{j}-\alpha_{j}^{*}\right)\phi \left(x_{j}\right). \end{array}$$

In (20), the parameter *α* and *α*^∗^ represent the nonzero value, often called Lagrange relaxation factor. Thus, the eventual output is obtained as

(21) $$\begin{array}{c} Y^{\prime }=\overset{l}{\underset{j=1}{\sum }}\left(\alpha_{j}-\alpha_{j}^{*}\right)\phi \left(x_{j}\right)*\phi \left(x\right)+b=\overset{l}{\underset{j=1}{\sum }}\left(\alpha_{j}-\alpha_{j}^{*}\right)*K\left(x_{j},x\right)+b. \end{array}$$

Here, *K*(*x*_*j*_, *x*) states the kernel function. In our proposed model, we applied the RBF kernel function to perform NoSQL-IA prediction or allied two-class (normal query and NoSQL-IA query) classification.

#### 5.6.3. Decision Tree (DT)

Decision tree (DT) being one of the most used association mining-based classifiers has evolved over the period due to its increasing significance and efficacy. It has emerged from the CART, ID3, C4.5, and C5.0 association rule mining models to serve classification tasks. Functionally, it originates at the root node, where applying the association rule in between the split condition, it divides the input features into multiple branches at each node of the tree. Subsequently, DT applies a factor called information gain ratio (IGR) for an individual branch of the tree. Functionally, once dividing the input data into multiple branches, it generates other nodes that subsequently branch-off into other nodes with corresponding instances. Thus, it resembles a tree structure with multiple branches. In other words, it resembles a binary tree with a parent node and multiple children's nodes, possessing left child and right child. Let the parent node, left child, and right child be *LC*_*d*_ and *RC*_*d*_, respectively. Now, with input feature *x*, the impurity measures *I*; we estimate the total samples in *P*_*d*_, *LC*_*d*_, and *RC*_*d*_; and decision tree method intends to enhance information gain using

(22) $$\begin{array}{c} Information\;Gain\;\left(P_{d}x\right)=I\left(P_{d}\right)-\frac{LC_{n}}{P_{n}}I\left(L.C_{d}\right)-\frac{RC_{n}}{P_{n}}I\left(R.C_{d}\right). \end{array}$$

In this method, the impurity measure *I* is calculated by applying three distinct approaches named, Gini-Index *I*_*G*_, Entropy *I*_*H*_, and classification error *I*_*E*_. These methods are mathematically defined as

(23) $$\begin{array}{c} I_{H}\left(n\right)=-\overset{c}{\underset{i=1}{\sum }}p\left(c\;|\;n\right)\log_{2}p\left(c\;|\;n\right), \end{array}$$

(24) $$\begin{array}{c} I_{G}\left(n\right)=1-\overset{c}{\underset{i=1}{\sum }}p{\left(c\;|\;n\right)}^{2}, \end{array}$$

(25) $$\begin{array}{c} I_{E}\left(n\right)=1-\max\left\{p\left(c\;|\;n\right)\right\}. \end{array}$$

In the above equations (23)–(24), the parameter *c* states the class(es), while a node is indicated by the term *n*. The ratio of *c* to *n* is given by *p*(*c* | *n*). In this manner, the proposed decision tree model labels each query as the normal query and NoSQL-IA query and labels each with “0” and “1,” respectively.

The article "Dynamic Data Infrastructure Security for Interoperable e-Healthcare Systems: A Semantic Feature-Driven NoSQL Intrusion Attack Detection Model" was retracted in 2024. Reasons: signs of a paper mill; suspected computer-generated content; unreliable results or conclusions; concerns about the data.

#### 5.6.4. Logistic Regression

In the at-hand two-class classification problem, the logistic regression (LOGR) algorithm performs regression over the input features by retaining feature instances as the independent variable while assigning their corresponding SQLIA probability as the dependent variable. To achieve it, we executed regression .

(26) $$\begin{array}{c} \text{logit}\left[\pi \left(\text{x}\right)\right]=\beta_{0}+\beta_{1}X_{1}+\beta_{2}X_{2}+\cdots \cdots .+\beta_{m}X_{m}. \end{array}$$

In (26), the function *logit*[*π*(*x*)] signifies the dependent variable while x_i_ states the independent variable. This function helped in transforming the dichotomous outputs by logit function resulting into varying *π*(*x*) in the range of 0 to 1 to −∞ to +∞. In (24), the parameter *m* states the total number of independent variables, while the NoSQL-IA probability is given by *π*. It estimated the probability of NoSQL-IA using

(27) $$\begin{array}{c} \pi \left(x\right)=\frac{e^{\beta_{0}+\beta_{1}X_{1}+\beta_{2}X_{2}+\cdots \cdots .+\beta_{m}X_{m}}}{1+e^{\beta_{0}+\beta_{1}X_{1}+\beta_{2}X_{2}+\cdots .+\beta_{m}X_{m}}}. \end{array}$$

#### 5.6.5. k-NN Algorithm

k-NN (k-nearest neighbor) is one of the most popular models that classify unlabeled observations or patterns by assigning it the class of the most similar labeled examples. The ease of implementation of k-NN makes it one of the most used classifiers for the different data mining and regression predictive tasks. Typically, k-NN algorithm applies Euclidean distance to estimate interattribute distance using

(28) $$\begin{array}{c} D\left(p,q\right)=\sqrt{{\left(p_{1}-q_{1}\right)}^{2}+{\left(p_{2}-q_{2}\right)}^{2}+{\left(p_{n}-q_{n}\right)}^{2}.} \end{array}$$

In (28), *p* and *q* are subjected to be compared with *n* features.

The efficiency of the k-NN algorithm depends on the value of *k* that decides how many neighbours can be selected for classification. Selection of an optimal *k* value helps achieve better performance. The large value of *k* minimizes the effect of a variance imposed by random error and forces it to be used with a low number of samples. The force maintaining an optimal balance between performance and computation (by selecting the optimal *k* value) depends on maintaining a better balance between overfitting and underfitting. In most of the existing methods, authors assigned the value of *k* as the square root of the number of instances in the training data; however, its efficacy for large-scale data with varying patterns cannot be guaranteed. In some works, *k* is assigned on the basis of the sample size by employing the cross-validation concept, however, at the cost of increased computation and time. To alleviate such problems, in this paper, a concept called *kTree* learning was applied, which helped us learn different *k* values for the different training samples. For training, *kTree* at first performs learning the optimal value of *k* for all data samples by applying the sparse reconstruction method. Subsequently, it constructs a decision tree (here we call *kTree*) using training samples and the learned optimal *k* values. During testing, *kTree* model outputs the value of *k* swiftly for each data (testing data) sample, which is then followed by *k* − *NN* classification using learned optimal *k* value and data training. Eventually, the proposed *k* − *NN* model classifies each query as a NoSQL-IA query and normal query and labels them with 1 and 0, respectively.

The article "Dynamic Data Infrastructure Security for Interoperable e-Healthcare Systems: A Semantic Feature-Driven NoSQL Intrusion Attack Detection Model" was retracted in 2024. Reasons: signs of a paper mill; suspected computer-generated content; unreliable results or conclusions; concerns about the data.

#### 5.6.6. AdaBoost

AdaBoost falls under the category of ensemble learning method designed as an adaptive bootstrap classifier. As the name indicates, it is called adaptive boosting as the learning weight parameters are reinforced for each instance, where it assigns higher weights to the wrongly classified data elements or instances. Functionally, being a meta-estimator, it is initiated by fitting a classifier deployed over the original datasets. Subsequently, it fits supplementary replicas of the classifiers on the same data but in that it adjusts the weights of the wrongly classified instances. In this manner, the replicated classifiers focus more on complex classification cases. In this manner, a number of weak learners are transformed into the stronger learner and hence achieves more accurate performance than the classical standalone classifier. In this work, AdaBoost classifies each input query into two classes, NoSQL-IA query and the normal query, and assigns a label to each with 1 and 0, correspondingly.

#### 5.6.7. Random Forest (RF) Algorithm

Similar to the AdaBoost classifier, random forest (RF) algorithm is a kind of ensemble learning method. It embodies multiple tree-structured learners giving rise to a new ensemble learning environment. In the constituted tree-structures, each tree performs classification distinctly over the input instances and labels data with a vote of class category. In the case of data classes be *N*, then it selects a sample containing *N*  cases arbitrarily from the input feature vector. The selected sample is later employed as the training set to form a tree. With *M* input instances, it divides the input instances *m* to split the node, where the value of *m* remains fixed throughout the forest development. In this manner, each tree develops a large tree structure with multiple branches and subtrees. Typically, RF needs lower tuning parameters that make it superior to other methods like Naïve Bayes, k-NN, and DT. RF, being the bootstrapped learning model, is mathematically derived as

(29) $$\begin{array}{c} \left\{h\left(x,\theta_{k}\right),k=1,2,\cdots i\cdots \right\}. \end{array}$$

In (29), *h* states the RF classifier, while {*θ*_*k*_} is the arbitrary vector distributed uniformly where each tree provides a vote for the high likelihood class for an input instance *x*. The size of *θ* often depends on its use towards tree formation. RF algorithm employs a bootstrapped subset of training samples which helps to perform training over each tree throughout the forest. This process applies almost 70% of the training data, while the remaining data is applied as the out-of-bag (OOB) samples. The OOB samples are employed to perform cross-validation that helps achieve higher accuracy [30]. As stated, functionally, RF as an ensemble model houses *T* trees, and thus, during training, the DTs are independently formed onto the bootstrap training set by applying randomly selected data. Noticeably, this approach applies feature selection methods like bagging and random subspace algorithm. In the proposed RF model, DT is constituted by using the following approach.

- Choose the training sample by replacing it from the original training data S. In this work, OOB samples (30%), which are except the bootstrapped sample, are applied to estimate the misclassification error
- Select *M* ≤ *D* features randomly and select the best split by applying Gini-Index method
- Develop tree to the highest depth

Over the classification process, the input data *x* is classified by traversing each tree until it reaches the leaf-node. Subsequently, it results in the classification output with the decision function *h*, which is deployed to each leaf node. In this manner, the final class label *y* is obtained by choosing the class having the highest rank or the votes. The final output is defined as

(30) $$\begin{array}{c} y=\underset{c\in \left\{\right\}}{\text{argm}1,2,\cdots ,\text{Cax}}\overset{T}{\underset{t:h_{t}\left(x\right)=c}{\sum }}1. \end{array}$$

The article "Dynamic Data Infrastructure Security for Interoperable e-Healthcare Systems: A Semantic Feature-Driven NoSQL Intrusion Attack Detection Model" was retracted in 2024. Reasons: signs of a paper mill; suspected computer-generated content; unreliable results or conclusions; concerns about the data.

#### 5.6.8. Extra Tree Classifier (ETC)

Similar to the above-discussed AdaBoost and RF ensemble methods, ETC forms a set of unpruned DTs by applying top-down concept. However, unlike RF it applies random instance as well as cut-point selection when performing tree-split. ETC distinguishes itself from other tree-based ensemble learning algorithms in reference to two factors. The first is that it divides nodes by choosing cut-points arbitrarily and by using the complete training sample. To be noted, unlike ETC, RF algorithm applies a bootstrap replica of the DT to form tree structure. The second distinguishing fact is that the classified results of all the encompassing trees are joined together to yield the final prediction result by applying the maximum voting ensemble (MVE) concept. The prime motive behind ETC is that the overall randomization of the cut-point and instances with ensemble averaging minimizes the variance in comparison to the weaker randomization methods, as applied in other ensemble approaches like RF and AdaBoost. In addition, the use of original training data rather than the bootstrap replicas alleviates the likelihood of any probable classification bias. Consequently, it helps ETC to achieve higher accuracy.

The article "Dynamic Data Infrastructure Security for Interoperable e-Healthcare Systems: A Semantic Feature-Driven NoSQL Intrusion Attack Detection Model" was retracted in 2024. Reasons: signs of a paper mill; suspected computer-generated content; unreliable results or conclusions; concerns about the data.

Thus, the proposed model applied these algorithms distinctly toward two-class classification to classify each input query as a NoSQL-IA query and normal query and labels them as 1 and 0, respectively. Here, our key motive was to identify the best set of feature engineering methods and the classifier performing the best performance towards NoSQL-IA intrusion prediction for Interoperable e-Healthcare Infrastructure security. A detailed discussion of the overall simulation results and allied inferences is given in the subsequent section.

## 6. Results and Discussion

This research work mainly focused on developing a robust and highly efficient NoSQL-IA prediction model for interoperable e-Healthcare systems to support seamless and reliable services. Unlike SQLIA methods which are often developed based on certain predefined syntax structure learning or term-matching concepts, this model considered distributed dynamic data structure resembling NoSQL databases where the data can be in heterogeneous data format. The likelihood of data heterogeneity and unstructuredness can be severe in the case of interoperable e-Healthcare systems that often support NoSQL database systems or infrastructures. In such a complex operating environment, the likelihood of intrusion attacks can be more probable, which can cause data breaches, manipulation, and even ransomware kinds of attacks. On the other hand, detecting aforesaid adversaries over interoperable e-Healthcare infrastructures with the large number of users can be highly complex and almost infeasible with manual test approaches or classical black-box techniques. To address these challenges, it was inevitable to exploit the maximum possible latent or semantic information from queries for highly advanced machine learning-based prediction. Considering the aforesaid challenges and allied scope, in this work, we formulated NoSQL-IA prediction as a semantic feature learning and natural language programming (NLP) problem. In addition, recalling the fact that the efficacy of any machine learning-driven NLP model(s) depends on the feature superiority and classification (computing) environment, we focused our effort on improving features as well as the overall computing environment. Our overall research intended to identify the optimal set of features and allied computing environment that could provide optimal performance toward NoSQL-IA prediction. Though there is no significant effort made so far towards NoSQL-IA prediction; however, for different intrusion detection or allied NLP problem, authors have claimed different features and allied computing environments to have better performance. However, no effort is available which could generalize the optimal feature and allied computing models towards NoSQL-IA or other intrusion detection or prediction systems. Considering this fact, we applied multiple semantic feature extraction methods along with the different feature selection, resampling, and classification models. Here, the prime motive was to identify the best performing feature and corresponding computing environment (such as feature selection method, resampling method, and classification model) so as to provide an optimal NoSQL-IA prediction solution which would perform gate-level intrusion detection as well as within-database intrusion identification and classification.

The article "Dynamic Data Infrastructure Security for Interoperable e-Healthcare Systems: A Semantic Feature-Driven NoSQL Intrusion Attack Detection Model" was retracted in 2024. Reasons: signs of a paper mill; suspected computer-generated content; unreliable results or conclusions; concerns about the data.

To achieve it, at first, we prepared our own synthetic data in sync with a real-time interoperable e-Healthcare system. The prepared data comprised a total of 14454 queries or transaction traces with almost 1400 intrusion queries. Once collecting the raw heterogeneous input data, we processed for preprocessing by applying tokenization followed by stopping words removal. Subsequently, unlike classical SQL-IA methods that often use structural or syntax information to perform intrusion detection, we applied the well-known word-embedding concepts to extract semantic features from each query. Here, we employed a total of five different semantic feature extraction methods, including Count Vectorizer, TF-IDF, Word2Vec, CBOW, Skip Gram, and GLOVE. Here, our key motive was to identify the best performing feature which could enable more efficient and reliable NoSQL-IA prediction. Undeniably, aforesaid methods yield high-dimensional semantic features towards learning, however, at the cost of increased computation. To alleviate this problem, we applied five different kinds of feature selection methods, including Select-K-Best (SKB), PCA, WRST, VTFS, and combined hybrid feature (AF). Here, we intended to assess with what specific feature selection model the optimal set of feature vectors could be obtained to perform NoSQL-IA prediction. To be noted, the intrusion queries are merely 9.7% of the total queries or data size. In other words, in the considered dataset, almost 92.3% of the samples or feature instances are majority class (i.e., normal query), while merely 9.7% of the samples are intrusion queries (say, minority class). This, as a result, shows the case of the imbalanced dataset and hence directly training a machine learning model with this data can force machine learning to undergo skewed performance or false-positive outputs. To alleviate this problem, we performed a resampling method, where we applied three different kinds of resampling methods, including downsampling (DNS), upsampling (UPS), and SMOTE sampling. Thus, once resampling the input features, it applied Min–Max normalization that mapped each input feature element in the range of 0-1 and thus helped in alleviating any possibility of overfitting or convergence. Once normalizing the inputs (from each feature sets over varied feature selection and resampling), each feature vector was processed for two-class classification using different machine learning models that classify each input query as the normal query or NoSQL-IA query and label them with 0 and 1, respectively. More specifically, we applied Naïve Bayes (with multinomial kernel function) classifier, k-NN, logistic regression (LOGR), decision tree (DT), support vector machine (with radial basis function kernel SVMR), AdaBoost (ADAB), random forest (RF), Extra Tree Classifier (ETC), and XGBoost (XGB). To assess relative performance towards NoSQL-IA prediction, we estimated confusion matrix and measured classification accuracy, F-Measure and AUC performance for each input feature, feature selection methods, resampling methods, and eventual classification models. The key motive was to identify the best performing feature and corresponding computing environment for the NoSQL-IA system to be used for interoperable e-Healthcare services or systems. The overall proposed model was developed using the Anaconda Spark development platform, where the programs were developed in Python language and simulated over Microsoft Windows operating system, armored with 8 GB RAM and a 2.82 GHz processor. To assess efficacy of the overall proposed model, the performance characterization is done in two phases: intramodel characterization and intermodel characterization. The detailed discussion of the results obtained is given as follows:

The article "Dynamic Data Infrastructure Security for Interoperable e-Healthcare Systems: A Semantic Feature-Driven NoSQL Intrusion Attack Detection Model" was retracted in 2024. Reasons: signs of a paper mill; suspected computer-generated content; unreliable results or conclusions; concerns about the data.

### 6.1. Intramodel Characterization

The performance assessment for the simulated results and allied inferences for the different features, feature selection methods, resampling approaches, and classifiers is discussed in intramodel characterization. Here, we intended to identify the best set of semantic features and allied computing environments (i.e., feature selection, resampling, and classification method(s)) for the NoSQL-IA prediction task.

#### 6.1.1. Assessing Semantic Feature Efficacy

Since different feature extraction methods claim their superiority over others in analytics or even in intrusion detection systems, we examined the relative efficacy of the different feature extraction methods toward NoSQL-IA prediction. As already discussed in the previous section, this work employed a total of six different word-embedding concepts, including Count Vectorizer (COUTV), TF-IDF, CBOW, SKG, Word2Vec (W2V), and GLOVE. A confusion matrix is an nXn matrix; each row reflects the true classification of observation, and each column represents the anticipated classification (or vice versa). When looking at a confusion matrix, the number of correct classifications may be determined by looking at the values on the diagonal; a successful model will have high counts (diagonal) and low counts off the diagonal. Furthermore, analyzing the highest count, not on the diagonal, can reveal the model's struggle. These evaluations are used to find scenarios when the model's accuracy is high, yet it consistently misclassifies the same data. The ratio of accurately anticipated positive observations to the predicted positive observations is called “precision.” The ratio of accurately predicted positive observations to all positive observations in the actual positive class is called “recall.” The weighted average of precision and recall is the F1-Measure. As a result, this score considers both false positives and false negatives. Although it is not as intuitive as accuracy, F1 is frequently more advantageous than accuracy, especially if the class distribution is unequal. When false positives and false negatives have equivalent costs, accuracy works well. It is the best to look at precision and recall if false positives and false negatives are considerably different. These different semantic algorithms have distinct computing or feature vector representation and hence can have different efficacies towards NoSQL-IA prediction. Figures 3–5 present the prediction accuracy (%), F-Measure, and AUC performance by these feature extraction methods, respectively.

Observing Figure 3, it can easily be found that N-Skip Gram method and CBOW algorithm exhibits superior accuracy to other semantic approaches. More specifically, N-Skip Gram features exhibited an accuracy of 97.63%, followed by the CBOW feature (96.41%), Gensim Word2Vec (96.2%), COUTV (94.7%), TF-IDF (94.2%), and GLOVE (88.68%). This result reveals that being distributed and significantly heterogeneous (dynamic in nature) in nature, approaches such as TF-IDF and Count Vectorizer (COUTV) are less significant as these methods often exploit the number of occurrences of the tokens rather than the allied latent information. On the contrary, Word2Vec (W2V), N-Skip Gram (SKG), and CBOW exploit interconnected semantic feature information to derive numerous (feature-vector) representations. In this manner, these methods do not lose feature information that helps better training and hence higher accuracy (Figure 3). GLOVE, a Wikipedia-driven pretrained feature set too, has been found limited over the proposed synthetic data environment, where the data queries were obtained from the varied users with autonomous query feeds and entries. The disparity of trained feature elements and input query variables has resulted in reduced performance for GLOVE, affirming the fact that a pretrained model like GLOVE or even W2V is required to be properly trained with the input data rather than generic dictionary variables or tokens.

The article "Dynamic Data Infrastructure Security for Interoperable e-Healthcare Systems: A Semantic Feature-Driven NoSQL Intrusion Attack Detection Model" was retracted in 2024. Reasons: signs of a paper mill; suspected computer-generated content; unreliable results or conclusions; concerns about the data.

Figure 4 presents the F-Measure performance of the different feature extraction methods. Similar to the accuracy performance, as discussed above (Figure 3), SKG, W2V, and CBOW features have shown superior F-score or F-Measure, signifying efficient performance in terms of sensitivity (recall) and precision. It affirms their suitability for the NoSQL-IA prediction task, which can undergo class-imbalance conditions. These features (i.e., SKG, W2V, and CBOW) can perform reliably without undergoing any false-positive or skewed performance. Noticeably, F-Measure with SKG feature was observed as 0.962, followed by W2V (0.957), CBOW (0.949), TF-IDF (0.936), COUTV (0.933), and GLOVE (0.904). Similar to accuracy performance (Figure 3), GLOVE exhibited the minimal F-Measure performance, signifying its inferiority over the other word-embedding methods like SKG, W2V, and CBOW.  Figure 5 depicts AUC performance, where SKG has been found superior over the other methods or features with its AUC value of 0.976, though other word-embedding methods like W2V and CBOW too exhibited AUC of 0.973, and 0.971, respectively. TF-IDF feature exhibited an AUC of 0.969, followed by COUTV (0.951) and GLOVE (0.947).

An interesting fact is that amongst all six different features, SKG and Word2Vec semantic features exhibited a minimum outlier or deviation in performance than other approaches and hence can be stated as the superior method towards reliable NoSQL-IA prediction tasks. Therefore, either of SKG or Word2Vec method can be applied towards semantic feature-driven NoSQL-IA prediction task.

#### 6.1.2. Assessing Feature Selection Efficacy

In this work, we applied four different kinds of feature selection methods named Significant K-Best 9SKB), principal component analysis (PCA), Wilcoxon Rank Sum Test (WRST), and variance threshold feature selection (VTFS). In addition to these, we merged different features (i.e., COUTV, TF-IDF, CBOW, SKG, W2V, and GLOVE) together to generate a hybrid feature set named all features (AF). For these different selected features, the performance was characterized in terms of accuracy (Figure 6), F-measure (Figure 7), and AUC (Figure 8). Figure 6 reveals that amongst the different feature selection methods, WRST exhibits the superior accuracy performance (accuracy 95.7%). The other methods like VTFS and PCA feature too exhibit the accuracy of 95.2% and 94.6%, respectively. Significant predictor test (SKB), which exploits interelement correlation towards prediction, could achieve the accuracy of 92.7%, while the hybrid feature (say, AF) performed poor with the classification accuracy of merely 87.8%. This can be mainly because of feature heterogeneity and ambiguity over learning a gigantic feature element together. This result (Figure 6) reveals that WRST (and VTFS as well) can be well-suited for feature selection in NLP-driven NoSQL-IA prediction tasks.

The article "Dynamic Data Infrastructure Security for Interoperable e-Healthcare Systems: A Semantic Feature-Driven NoSQL Intrusion Attack Detection Model" was retracted in 2024. Reasons: signs of a paper mill; suspected computer-generated content; unreliable results or conclusions; concerns about the data.

Figure 7 shows F-Measure performance by the different feature selection methods. As depicted, similar to Figure 6, WRST, VTFS, and PCA have exhibited superior performance (WRST (0.956), PCA (0.951), and VTFS (0.948)) over other methods like SKB (0.927). It also confirms that the amalgamation of the different features together can force the model to undergo convergence or overfitting and hence can result in poor performance (AF-0.86).

Considering AUC performance over the different feature selection methods, the result (Figure 8) exhibits that the WRST method yields higher AUC (0.984) than other methods like (PCA (0.978), SKB (0.977), VTFS (0.972), and AF (0.941)), Noticeably, higher AUC affirms robustness of the method(s) towards prediction over nonlinear, heterogeneous, and imbalanced data environment like NoSQL-IA prediction system. It affirms that WRST feature selection can be a superior solution towards NoSQL-IA prediction.

#### 6.1.3. Assessing Feature Resampling

As already stated, the current NoSQL-IA prediction problem undergoes class imbalance, and hence, to alleviate it, we employed three different kinds of resampling methods: SMOTE, upsampling (UPS), and downsampling (DNS). The accuracy performance, as depicted in Figure 9, reveals that SMOTE sampling performs an accuracy of 96.4%, which is almost the same as UPS which exhibited a prediction accuracy of 96.32%, though DNS underwent reduced performance with an accuracy of 88.96%.

Considering F-Measure performance, the result (Figure 10) reveals that UPS and SMOTE perform similar approximate performance (F-measure 0.952), which is higher than the downsampling method DNS (0.875). A similar performance can be observed in Figure 11 as well, where UPS exhibited superior AUC (0.988) followed by SMOTE (0.983) and DNS (0.879). Noticeably, though upsampling (UPS) method has exhibited relatively better performance; however, the allied probability of skewed data cannot be universally eliminated. High upsampling might even skew the data and hence can give rise to the data imbalance. Therefore, in comparison to UPS, SMOTE sampling can be a better alternative for NoSQL-IA prediction.

The article "Dynamic Data Infrastructure Security for Interoperable e-Healthcare Systems: A Semantic Feature-Driven NoSQL Intrusion Attack Detection Model" was retracted in 2024. Reasons: signs of a paper mill; suspected computer-generated content; unreliable results or conclusions; concerns about the data.

#### 6.1.4. Assessing NoSQL-IA Classification

In this work, we exploited the relative performance of the different machine learning algorithms toward NoSQL-IA prediction. The relative performance outputs by the different machine learning algorithms are given in Figures 12–14. The depth assessment revealed that the average accuracy by Naïve Bayes (multinomial kernel function) method was 96.98%, while k-NN could achieve the average accuracy of 74.37%. The other methods like DT, LOGR, SVM, ADAB, RF, ETC, and XGB exhibited the prediction accuracy of 87.61%, 92.37%, 88.04%, 91.50%, 98.86%, 89.51%, and 93.47%, respectively. The performance assessment reveals that amongst the different machine learning models, the random forest (RF) method exhibited superior performance with the highest accuracy of 98.86%.

The average F-Measure performance by the different machine learning classifiers exhibited that similar to the accuracy output (Figure 12), the RF classifier exhibited the highest F-Measure of 0.974. The other methods like NB, k-NN, DT, LOGR, SVM, ADAB, ETC, and XGB could exhibit the average F-Measure of 0.89, 0.794, 0.90, 0.933, 0.888, 0.936, 0.867, and 0.911, respectively. Though the F-Measure performance by these algorithms is higher than the hypothetical scale of 0.6; however, the results (Figures 12 and 13) affirm that RF method can be vital towards NoSQL-IA prediction system, where it can yield higher accuracy than the other standalone methods. To be noted, RF being the bootstrapped decision tree has confirmed its superiority over the standalone DT method and hence performs in sync with the development goal (i.e., to achieve better performance than the classical or standalone DT algorithm).

Figure 14 shows AUC performance by the different machine learning classifiers towards NoSQL-IA prediction. The average AUC by NB, k-NN, DT, LOGR, SVMR, ADAB, RF, ETC, and XGB was obtained as 0.958, 0.846, 0.923, 0.956, 0.905, 0.975, 0.987, 0.920, and 0.954, respectively. Observing result, it can be found that the RF algorithm performs better AUC (0.987) than other methods toward NoSQL-IA prediction.

Similar to the above statement, the majority of NLP problems or classification problems hypothesize that a model with AUC of more than 0.66 (sometime 0.6) is supposed to be efficient towards analytics problems; though all classifiers have achieved higher AUC, and it can be used for real-time computation, the relative performance confirms the robustness of RF over other methods. The overall classification or allied prediction results (Figures 12–14) confirm that RF can be a superior ensemble learning model for NoSQL-IA prediction.

The article "Dynamic Data Infrastructure Security for Interoperable e-Healthcare Systems: A Semantic Feature-Driven NoSQL Intrusion Attack Detection Model" was retracted in 2024. Reasons: signs of a paper mill; suspected computer-generated content; unreliable results or conclusions; concerns about the data.

Considering overall performance, it can easily be found that towards NoSQL-IA prediction task, the use of word-embedding methods like N-Skip Gram and Word2Vec can be a suitable semantic feature, while WRST can be a suitable and lightweight feature selection approach. WRST can not only retain significant features, but can also reduce data search space so as to improve overall NoSQL-IA prediction. It makes it suitable towards real-time applications demanding a swift and reliable analytics platform for intrusion detection. Similarly, in sync with aforesaid Word2Vec (word-embedding) features and corresponding WRST feature selection, the use of SMOTE sampling can help alleviate any possible data-imbalance problem. It can help improve overall accuracy and reliability even under class-imbalanced conditions. Finally, the SMOTE resampled feature vector (post-normalization) can be classified using the RF algorithm, a bootstrapped ensemble learning classifier to yield optimal and most efficient (say, reliable and highly accurate) NoSQL-IA prediction model for real-time intrusion detection in interoperable e-Healthcare system of services.

### 6.2. Intermodel Characterization

In this section, the relative performance assessment is done with reference to the existing methods. This is the matter of fact that a few efforts have been made towards NoSQL-IA detection; however, the extensive survey and analysis identified a few recent works including the efforts in [41, 42]. Authors in [41] focused on intrusion detection in distributed dynamic datasets with multiple users. The data construction proposed in [41] was followed in this work, where considering heterogeneous data nature and distributed dynamically in nature MongoDB database was considered. To be noted, amongst NoSQL databases, MongoDB is a kind of document-based database, while other NoSQL databases like Couchbase, Dynamo, Redis, Riak, and OrientDB store data in the form of keys and values. Similarly, Cassandra, HBase, vertical stores data in column-oriented architecture, Neo4J, Allegro Graph, and Stardog are also the kind of NoSQL databases that store data in the form of graphs. Considering the heterogeneous nature of interoperable healthcare datasets and allied characteristics [44], we considered MongoDB as the test dataset, where the data is in the form of a document and hence applying word-embedding was easier over the continuous documents or allied corpus. Thus, considering the similarity of data and motive, we compared the performance of our proposed NoSQL-IA prediction model with [41, 42]. Comparison model one [41] has applied One-class SVM (OC-SVM), whereas model two [42] has applied the Bayesian network as K2 algorithm (simulated onto WEKA tool) for intrusion detection over NoSQL data. Noticeably, both these datasets employed MongoDB data structure which is quite common in interoperable system designs. The relative performance assessment revealed that the average AUC performance in [41] was 0.959, which is lower in comparison to our proposed NoSQL-IA prediction model, which exhibited an average AUC of 0.981 with RF classifier. Interestingly, with an SVM classifier, our proposed NoSQL-IA model could achieve the average AUC of 0.905, which is lower than both our proposed RF-based prediction as well as the existing OC-SVM-based intrusion detection model [41]. It signifies that the use of ensemble learning methods like RF, XGB, and ETC can be superior to the standalone classifier for NoSQL intrusion detection and classification. Authors in [42] applied the K2 algorithm for intrusion detection, where the different NoSQL datasets like KDD99, DARPA1998, and DARPA1999 were applied as input data for intrusion detection. Though aforesaid datasets belong to NoSQL category, however, it differs from the real-time intrusion cases like camouflage query-driven attack, bots driven attack, mimicking attacks, etc. To represent their model as a NoSQL system, the authors merged aforesaid datasets (i.e., KDD99, DARPA1998, and DARPA1999) to generate a MongoDB dataset for further analysis. To improve feature efficiency, authors [42] applied factorial multiple correspondence analysis (FMCA) method. On the contrary, in our proposed model, we employed multiple highly robust statistical analysis approaches to retain the most significant features while guaranteeing their semantic feature retention. The data considered in [42] encompassed multiple datasets and hence possessed different attack conditions. Considering this fact, we averaged the accuracy performance of [42] and found that the average intrusion detection accuracy of their model was 92.37%. On the contrary, the average NoSQL-IA prediction accuracy by our proposed model (with RF classifier) is 98.86%. The relative performance with the existing methods [41, 42] reveals that the proposed NoSQL-IA prediction approach with Word2Vec word-embedding (semantic) features processed with WTFS feature selection, SMOTE sampling, Min-Max normalization, and RF classification yields better performance than any other existing NoSQL-IA prediction or classification approaches. Authors in [43] applied different machine learning methods towards intrusion detection in MongoDB-driven analytics. The recall and precision performance revealed that the highest recall or sensitivity with RF was 0.9137, followed by k-NN (0.8756), DT (0.8725), and Naïve Bayes (NB) (0.8720). Similar simulation results were obtained in the form of precision parameters. However, it indicates lower performance than the proposed NoSQL-IA prediction model. Recall and precision are the key driving elements of F-score or F-Measure, and therefore, higher value of F-Measure (0.937) of the proposed model indicates the higher value of precision and recall. It indicates superior performance by our proposed RF-driven NoSQL-IA prediction performance. Thus, observing overall results and allied inferences, it can be stated that the proposed NoSQL-IA model exhibits superior performance to the other state-of-the-art methods. The research conclusion and allied inferences are given in the subsequent section.

The article "Dynamic Data Infrastructure Security for Interoperable e-Healthcare Systems: A Semantic Feature-Driven NoSQL Intrusion Attack Detection Model" was retracted in 2024. Reasons: signs of a paper mill; suspected computer-generated content; unreliable results or conclusions; concerns about the data.

## 7. Conclusion

This paper mainly focused on achieving an optimal set of computing environments for highly efficient intrusion detection systems for interoperable e-Healthcare systems. In sync with the aforesaid motive, this research made an effort to address the key real-time problems, including data heterogeneity, minimal intelligibility over interoperable systems having multiple stakeholders, class imbalance, and diversified performance by the different machine learning models towards intrusion detection (and classification) in dynamic data structures or NoSQL databases. The research is limited to constructing the optimized semantic feature-based IDS model as part of NoSQL-IA. The study can be further extended to explore the possibility of keeping the model optimal with periodic retraining. The case of asynchronous IDA execution can be considered at the server level. Summarily, this work contributed a first of its kind NoSQL-IA detection and classification system to be used for interoperable e-Healthcare services. To address data heterogeneity over an interoperable multistakeholder environment, the proposed model employed the semantic feature learning concept BERT (Bidirectional Encoder Representations from Transformers) which is an open-source machine learning framework for natural language processing (NLP) that uses surrounding text to establish context to help computers learn the meaning of ambiguous language in the text data. There is a possibility of exploring the BERT pretrained framework for text classification considering the deployment environment and model serving the architecture as future scope of work. Since different algorithms claim their superiority over others in semantic feature retention, this work applied four different well-known algorithms, including Word2Vec, GLOVE, TF-IDF, and CBOW, for feature extraction. Here, the motive was to identify the best performing semantic features for NoSQL-IA attack detection. The topic model Latent Dirichlet Allocation (LDA) is used to classify text in a document to a particular topic. It creates a Dirichlet distribution-based topic per document and word per topic model. The author in [55] discussed LDA and Word2Vec as a hybrid document feature extraction method. They obtain an F1 score of 0.8 for a topic of 250. Our input data is not of abstract group nature, and hence, this method shall not fit into the study's scope. Applying the aforesaid semantic feature extraction method imposes data search space to reduce computational overheads in real-time; the proposed model applied feature selection methods like PCA, WRST significant predictor test, Select-K-Best, and VTFS algorithms over the extracted features. The purpose of these feature selection methods was to reduce computational overhead so as to cope with the run-time demands. Subsequently, it applied resampling methods, which helped in alleviating any class-imbalance problem that can impose any machine learning model to undergo false-positive or skewed performance. More specifically, this work applied upsampling, random sampling, and SMOTE-ENN methods. Moreover, the use of Min–Max normalization helped alleviate the overfitting problem to support better training. The proposed model was trained over each input query and allied label, which helped in performing two-class classification, where it predicts each input query as a normal query or intrusion (or NoSQL-IA attack). To identify the best classification environment towards NoSQL-IA prediction, this work employed Naïve Bayes, decision tree, k-NN, gradient boosting, random forest, and XG-Boost algorithms. The depth performance assessment of the developed NoSQL-IA model revealed that the use of SKG, Word2Vec word-embedding features, followed by SMOTE resampling, and Random Forest classification can yield the most accurate and reliable performance towards intrusion prediction under heterogeneous interoperable e-Healthcare systems. The overall performance reveals that the proposed SKG semantic feature-driven model with WRST feature selection, SMOTE resampling, Min–Max normalization, and RF classifier-based prediction yields a superior accuracy of 98.86%, F-Measure of 0.936, and AUC of 0.987. The aforesaid feature (i.e., SKG word-embedding or Word2Vec) with a computational environment (WRST as feature selection, SMOTE as resampling method, and Min–Max normalization followed by Random Forest ensemble classification) can yield optimal performance towards NoSQL-IA prediction in interoperable e-Healthcare systems. Since the proposed model was designed especially in sync with heterogeneous input queries and semantic features, its intelligibility affirms its suitability for real-time intrusion detection in e-Healthcare services.

The article "Dynamic Data Infrastructure Security for Interoperable e-Healthcare Systems: A Semantic Feature-Driven NoSQL Intrusion Attack Detection Model" was retracted in 2024. Reasons: signs of a paper mill; suspected computer-generated content; unreliable results or conclusions; concerns about the data.

## Figures and Tables

**Figure 1:** Permissions for the killing process.

**Figure 2:** Setup for normal and intrusion transaction trace(s) generation towards distributed dynamic database generation and NoSQL-IA prediction.

**Figure 3:** Accuracy of the different semantic features towards NoSQL-IA prediction.

**Figure 4:** F-Measure of the different semantic features towards NoSQL-IA prediction.

**Figure 5:** AUC of the different semantic features towards NoSQL-IA prediction.

**Figure 6:** Accuracy with the different features selection methods towards NoSQL-IA prediction.

**Figure 7:** F-Measure with the different features selection methods towards NoSQL-IA prediction.

**Figure 8:** AUC with the different features selection methods towards NoSQL-IA prediction.

**Figure 9:** Accuracy (%) with the different features resampling methods towards NoSQL-IA prediction.

**Figure 10:** F-Measure with the different features resampling methods towards NoSQL-IA prediction.

**Figure 11:** AUC with the different features resampling methods towards NoSQL-IA prediction.

**Figure 12:** Accuracy with the different classifiers towards NoSQL-IA prediction.

**Figure 13:** F-Measure with the different classifiers towards NoSQL-IA prediction.

**Figure 14:** AUC with the different classifiers towards NoSQL-IA prediction.

**Code 1:** 

**Table 1:** Training data structure.

Input feature	Resampling	Normalized feature
*Feat*_*Word*2*Vec*_*NNorm*	(*Feat*_*Word*2*Vec*_*NNorm*)_*UpSampling*	*Norm*(*Feat*_*Word*2*Vec*_*NNorm*)_*UpSampling*
	(*Feat*_*Word*2*Vec*_*NNorm*)_*DownSampling*	*Norm*(*Feat*_*Word*2*Vec*_*NNorm*)_*DownSampling*
	(*Feat*_*Word*2*Vec*_*NNorm*)_*SMOTESampling*	*Norm*(*Feat*_*Word*2*Vec*_*NNorm*)_*SMOTESampling*
*Feat*_*Word*2*Vec*_*CBOW*	(*Feat*_*Word*2*Vec*_*CBOW*)_*UpSampling*	*Norm*(*Feat*_*Word*2*Vec*_*CBOW*)_*UpSampling*
	(*Feat*_*Word*2*Vec*_*CBOW*)_*DownSampling*	*Norm*(*Feat*_*Word*2*Vec*_*CBOW*)_*DownSampling*
	(*Feat*_*Word*2*Vec*_*CBOW*)_*SMOTESampling*	*Norm*(*Feat*_*Word*2*Vec*_*CBOW*)_*SMOTESampling*
*Feat*_*GLOVE*	(*Feat*_*GLOVE*)_*UpSampling*	*Norm*(*Feat*_*GLOVE*)_*UpSampling*
	(*Feat*_*GLOVE*)_*DownSampling*	*Norm*(*Feat*_*GLOVE*)_*DownSampling*
	(*Feat*_*GLOVE*)_*SMOTESampling*	*Norm*(*Feat*_*GLOVE*)_*SMOTESampling*
*Feat*_*TF* − *IDF*	(*Feat*_*TF* − *IDF*)_*UpSampling*	*Norm*(*Feat*_*TF* − *IDF*)_*UpSampling*
	(*Feat*_*TF* − *IDF*)_*DownSampling*	*Norm*(*Feat*_*TF* − *IDF*)_*DownSampling*
	(*Feat*_*TF* − *IDF*)_*SMOTESampling*	*Norm*(*Feat*_*TF* − *IDF*)_*SMOTESampling*
*Feat*_*W*2*V*	(*Feat*_*W*2*V*)_*UpSampling*	*Norm*(*Feat*_*W*2*V*)_*UpSampling*
	(*Feat*_*W*2*V*)_*DownSampling*	*Norm*(*Feat*_*W*2*V*)_*DownSampling*
	(*Feat*_*W*2*V*)_*SMOTESampling*	*Norm*(*Feat*_*W*2*V*)_*SMOTESampling*
*Feat*_*COUTV*	(*Feat*_*COUTV*)_*UpSampling*	*Norm*(*Feat*_*COUTV*)_*UpSampling*
	(*Feat*_*COUTV*)_*DownSampling*	*Norm*(*Feat*_*COUTV*)_*DownSampling*
	(*Feat*_*COUTV*)_*SMOTESampling*	*Norm*(*Feat*_*COUTV*)_*SMOTESampling*

The article "Dynamic Data Infrastructure Security for Interoperable e-Healthcare Systems: A Semantic Feature-Driven NoSQL Intrusion Attack Detection Model" was retracted in 2024. Reasons: signs of a paper mill; suspected computer-generated content; unreliable results or conclusions; concerns about the data.

## Data Availability

Data will be made available on request from the corresponding author.
